The article "Dietary Plant Polyphenols as the Potential Drugs in Neurodegenerative Diseases: Current Evidence, Advances, and Opportunities" was published in 2022. Journal: Oxid Med Cell Longev.

# Dietary Plant Polyphenols as the Potential Drugs in Neurodegenerative Diseases: Current Evidence, Advances, and Opportunities

**DOI:** 10.1155/2022/5288698

**Published:** 2022-02-21

**Authors:** Lu Yan, Min-Song Guo, Yue Zhang, Lu Yu, Jian-Ming Wu, Yong Tang, Wei Ai, Feng-Dan Zhu, Betty Yuen-Kwan Law, Qi Chen, Chong-Lin Yu, Vincent Kam-Wai Wong, Hua Li, Mao Li, Xiao-Gang Zhou, Da-Lian Qin, An-Guo Wu

**Affiliations:** ^1^Sichuan Key Medical Laboratory of New Drug Discovery and Druggability Evaluation, Luzhou Key Laboratory of Activity Screening and Druggability Evaluation for Chinese Materia Medica, School of Pharmacy; Education Ministry Key Laboratory of Medical Electrophysiology, College of Preclinical Medicine, Southwest Medical University, Luzhou 646000, China; ^2^State Key Laboratory of Quality Research in Chinese Medicine, Macau University of Science and Technology, Taipa, Macau SAR, China; ^3^Department of Nursing, Affiliated Hospital of Southwest Medical University, Luzhou, China

## Abstract

Neurodegenerative diseases, including Alzheimer's disease (AD), Parkinson's disease (PD), and Huntington's disease (HD), are characterized by the progressive degeneration of neurons. Although the etiology and pathogenesis of neurodegenerative diseases have been studied intensively, the mechanism is still in its infancy. In general, most neurodegenerative diseases share common molecular mechanisms, and multiple risks interact and promote the pathologic process of neurogenerative diseases. At present, most of the approved drugs only alleviate the clinical symptoms but fail to cure neurodegenerative diseases. Numerous studies indicate that dietary plant polyphenols are safe and exhibit potent neuroprotective effects in various neurodegenerative diseases. However, low bioavailability is the biggest obstacle for polyphenol that largely limits its adoption from evidence into clinical practice. In this review, we summarized the widely recognized mechanisms associated with neurodegenerative diseases, such as misfolded proteins, mitochondrial dysfunction, oxidative damage, and neuroinflammatory responses. In addition, we summarized the research advances about the neuroprotective effect of the most widely reported dietary plant polyphenols. Moreover, we discussed the current clinical study and application of polyphenols and the factors that result in low bioavailability, such as poor stability and low permeability across the blood-brain barrier (BBB). In the future, the improvement of absorption and stability, modification of structure and formulation, and the combination therapy will provide more opportunities from the laboratory into the clinic for polyphenols. Lastly, we hope that the present review will encourage further researches on natural dietary polyphenols in the treatment of neurodegenerative diseases.

The article "Dietary Plant Polyphenols as the Potential Drugs in Neurodegenerative Diseases: Current Evidence, Advances, and Opportunities" was published in 2022. Journal: Oxid Med Cell Longev.

## 1. Introduction

Neurodegenerative diseases, including Alzheimer's disease (AD), Parkinson's disease (PD), Huntington's disease (HD), amyotrophic lateral sclerosis (ALS), and multiple sclerosis (MS), are a group of incurable heterogeneous diseases. They are characterized by the gradual degeneration of the function and structure of neurons and overactivation of microglia in the central nervous system (CNS) [1]. To date, the accurate molecular mechanisms related to the pathogenesis and progression of neurodegenerative diseases are not well elucidated [2]. Although each neurodegenerative disease exhibits the respective pathological features, they also share some common molecular mechanisms, such as the aggregation of misfolded proteins, oxidative damage, mitochondrial dysfunction, DNA damage, neuroexcitotoxicity, biometal dyshomeostasis, neurotrophic impairment, and neuroinflammatory responses [3, 4]. Among them, the aggregated misfolded proteins have become the pathological hallmarks in many neurodegenerative diseases. For example, the extracellular deposition of amyloid-*β* (A*β*) fibrils and intracellular hyperphosphorylated Tau are found in the brain of AD. In addition, Lewy bodies containing *α*-synuclein, mutant huntingtin (mHtt), mutant superoxide dismutase 1 (SOD1), and TAR DNA-Binding Protein 43 (TDP-43) are closely associated with the pathogenesis of PD, HD, and ALS, respectively [5]. It is known to us that these misfolded proteins are increasingly accumulated with ageing and induce oxidative stress by generating excessive reactive oxygen species (ROS) and reactive nitrogen species (RNS), which is accompanied by mitochondrial dysfunction, DNA damage, neuroexcitotoxicity, and ultimately neuronal death [6]. In addition, neuroinflammation plays a critical role in the early onset and late-stage of neurodegenerative diseases [7]. Microglia known as the resident macrophage cells in the brain are chronically activated by the Pathogen-Associated Molecular Patterns or Danger-Associated Molecular Patterns (PAMPs/DAMPs), such as misfolded protein aggregates, bacteria, viruses, lipopolysaccharides (LPS), and many environmental toxins. Then, the sustained activated microglia subsequently release several cytokines and induce proinflammatory responses [8]. Therefore, neuronal death and microglial overactivation are two major indicators for the pathological development and process of neurodegenerative diseases. Emerging evidence indicates that the autophagy-lysosome pathway (ALP) and the ubiquitin-proteasome system (UPS) are two important processes that facilitate the clearance of misfolded proteins and damaged or unnecessary organelles, such as mitochondria [9]. At the early onset of neurodegenerative diseases, ALP and UPS acting as collaborators play protective roles in the degradation of toxin misfolded proteins, resistance to oxidative stress, and suppression of neuroinflammation [10, 11]. However, the normal function of ALP and UPS is impaired with ageing by the increasingly accumulated misfolded proteins and toxins [12, 13]. In this review, we summarized the current well-studied molecular mechanisms closely associated with the development of neurodegenerative diseases, including the aggregation of misfolded proteins, oxidative damage, mitochondrial dysfunction, DNA damage, excitotoxicity, biometal dyshomeostasis, and neuroinflammatory responses. However, the molecular mechanism of neurodegenerative diseases is still in its infancy and requires further in-depth investigations.

The article "Dietary Plant Polyphenols as the Potential Drugs in Neurodegenerative Diseases: Current Evidence, Advances, and Opportunities" was published in 2022. Journal: Oxid Med Cell Longev.

At present, there are currently many drugs developed and approved for the improvement of the symptoms of patients with neurodegenerative diseases in the clinical, but few of them can cure these diseases. More seriously, there might have side effects that appeared owing to the long-term use. In addition, many drugs, such as bapineuzumab, gantenerumab, and solanezumab, were recently declared failures during the clinical trial [14, 15]. Therefore, the accurate molecular mechanism and discovery of targeted drugs for the treatment of neurodegenerative diseases are still urgent and attract more and more attention [16]. In this review, we summarized the main current therapies and their mechanisms of action, neuroprotective effects, and limitations in various neurodegenerative diseases (Table 1). In view of the diversity of pathogenic mechanisms, the combinational therapies or the discovery and development of drugs with multitargets bring new hope for the treatment of neurodegenerative diseases. Therefore, more and more attentions are paid to natural medicine such as traditional Chinese medicines (TCMs) with multicompounds, multitargets, and multieffect properties. TCMs originating from natural products have a 2000-year history of treating diseases in China and have been proved to be safe and effective. To date, various kinds of bioactive compounds, including alkaloids, polyphenols, and saponins, are isolated and identified from natural plants. Among them, polyphenols, an important type of natural product, are mainly widely distributed in natural dietary plants. They are commonly divided into flavonoids and nonflavonoids which are subclassified into phenolic acids, stilbenes, lignans, curcuminoids, and coumarins. The modern pharmacological studies demonstrate that these polyphenols exhibit potential neuroprotective effects including the inhibition of neuronal death and the attenuation of neuroinflammatory responses in vitro and in vivo [17]. In this review, we summarized the research advances about the neuroprotective effect of the most widely reported dietary plant polyphenols in various cellular and animal models of neurodegenerative diseases. In addition, we discussed the current clinical study and application of polyphenols and the factors that result in low bioavailability. In the future, we hope that the improvement of absorption and stability, the modification of structure and formulation, and the combination therapy will provide more opportunities from the laboratory into the clinic for polyphenols. The present review will aid the researchers to know the research advances of polyphenols in neurodegenerative diseases. Lastly, we hope further researches will be encouraged for natural dietary polyphenols in the treatment of neurodegenerative diseases.

The article "Dietary Plant Polyphenols as the Potential Drugs in Neurodegenerative Diseases: Current Evidence, Advances, and Opportunities" was published in 2022. Journal: Oxid Med Cell Longev.

## 2. The Common Molecular Mechanisms of Neurodegenerative Diseases

### 2.1. Aggregation of Misfolded Proteins

The aggregation of misfolded proteins is recognized to be the common pathological feature of neurodegenerative diseases, such as A*β* and hyperphosphorylated Tau in AD, mutant *α*-synuclein in PD, and mHtt in HD, as well as SOD1 and TDP-43 in ALS [5, 34, 35] (Figure 1). It is known to us that ALP and UPS are two major intracellular elimination pathways for the clearance of these neurotoxic proteins in neurons and other cells in the brain [9, 36–38]. In the early onset of neurodegenerative disease, these toxic misfolded proteins are degraded via ALP and UPS pathways or effectively engulfed by microglia and astrocytes under normal physiological conditions. However, there is a growing body of studies showing that these misfolded protein aggregates are increasingly accumulated with ageing, accompanied by dysregulated or impaired ALP and UPS, which is implicated in the late stage of various neurodegenerative diseases [39]. Lastly, the normal function of neurons is becoming lost, and the microglia are overactivated, which ultimately results in neuronal death and proinflammatory responses [40] (Figure 1). For example, many accumulated autophagosomes and autophagic vesicles in the brain of AD patients are observed at the late stage of autophagy flux under immunoelectron microscopy [41]. In addition, autophagy is activated in the brain cells of AD patients and APP/PS1 mice. However, autophagy is impaired with ageing as revealed by the accumulation of A*β*-containing autophagic vesicles [42]. Therefore, autophagy plays a protective mechanism that fights against toxic protein-induced neuronal death and neuroinflammation at the early stage of AD, while the normal function of autophagy is impaired by the overgenerated toxic misfolded proteins (e.g., A*β* and Tau). In PD, emerging evidence indicates that the accumulation of mutant genes, including *α*-synuclein, Parkin, and ubiquitin carboxy-terminal hydrolase L1 (UCHL-1), is closely associated with the dysfunction of ALP and UPS [43]. At the early stage of PD, autophagy participates in the clearance of misfolded proteins, damaged mitochondria, and generated ROS. However, autophagy is impaired in the brain of PD toxin-induced animals or transgenic mice with PD. For instance, the mRNA level of ubiquitinated *α*-synuclein is significantly increased in the brain of 1-methy-4-phenyl-1,2,3,6-tetrahydropyridine- (MPTP-) induced mice [44]. In addition, the impaired lysosome is accompanied by the accumulation of *α*-synuclein in mice which are chronically injected with probenecid and MPTP [45]. There is a growing body of evidence showing that UPS plays an important role in the degradation of soluble mHtt, but almost 90% of long-lived or large aggregated proteins such as mHtt can only be degraded via ALP [46]. For example, rapamycin, a potent autophagy inducer, significantly accelerates the autophagic degradation of mHtt, while autophagy inhibitors including 3-methyladenine (3-MA) and bafilomycin A1 attenuate the effect of rapamycin [47, 48]. Taken together, the aggregation of misfolded proteins is the pathological hallmarks of neurodegenerative diseases, while ALP and UPS act as a protective mechanism that timely clears the misfolded protein aggregates to maintain cellular homeostasis at the early stage of neurodegenerative diseases. However, misfolded proteins are increasingly accumulated with ageing, which dysregulates the normal functions of ALP and UPS [49]. Therefore, the discovery of ALP or UPS enhancers that target the clearance of misfolded proteins and damaged organelles is recognized to be a promising therapeutic strategy for neurodegenerative diseases.

The article "Dietary Plant Polyphenols as the Potential Drugs in Neurodegenerative Diseases: Current Evidence, Advances, and Opportunities" was published in 2022. Journal: Oxid Med Cell Longev.

### 2.2. Oxidative Stress

In general, oxidative stress is caused by the imbalance between oxidation and antioxidation when the free radicals including superoxide anion radical and hydroxyl radical are overgenerated and cannot be cleared timely and effectively [50, 51]. Oxidative stress is currently implicated in various diseases, such as neurodegenerative diseases, ageing, atherosclerosis, and cancers. It is characterized by mitochondrial dysfunction and abnormal accumulation of transition metals, which causes mitochondrial DNA (mtDNA) mutations, changes in membrane permeability, calcium dyshomeostasis, lipid oxidation generation, and protein carbonylation [52]. Emerging evidence indicates that the brain cells are more susceptible to oxidative damage owing to the high oxygen consumption and the weak antioxidant defence ability [53]. The mechanistic studies demonstrate that oxidative stress is a critical inducer of neuronal death and neuroinflammation in neurodegenerative diseases [54]. It is reported that the misfolded protein aggregates (A*β*, Tau, a-synuclein, mHtt, *etc.*) damage the normal function of mitochondria, which then induces the generation of amounts of ROS [6, 55]. In turn, excessive ROS levels promote the aggregation of the pathological proteins [56]. For example, oxidative stress is reported to promote A*β* deposition, Tau hyperphosphorylation, and the subsequent loss of synapses and neurons in AD [57] and also induce the degeneration of dopaminergic neurons in the substantia nigra of PD brain [58, 59]. In addition, oxidative stress also overactivated microglia and induces neuroinflammation [60], while neuroinflammation further aggravates the accumulation of misfolded proteins and induces oxidative stress [61]. Collectively, a vicious circle among oxidative stress, misfolded proteins, neuronal death, and neuroinflammation is formed, which collaboratively induces the onset of neurodegenerative diseases and accelerates the progress and development of pathology. At present, several studies indicate that the activation of Kelch-like ECH-associated protein 1/nuclear factor erythroid 2-related factor 2/antioxidant response element (Keap1/Nrf2/ARE) pathway has a certain neuroprotective effect in numerous cellular and animal models of neurodegenerative diseases. However, there is limited clinical evidence showing that Nrf2 activation is a clinical target in neurodegenerative disease except for MS [62, 63] (Figure 2). Thus, more clinical studies are needed to be carried out for the validation and confirmation of the neuroprotective effect of Nrf2 target and its activators. Collectively, the discovery of antioxidants targeting the inhibition of oxidative stress to suppress neuronal death and neuroinflammation is an effective therapeutic strategy for neurodegenerative diseases.

### 2.3. Mitochondrial Dysfunction

Mitochondria, membrane-bound organelles located in the cytoplasm of almost all eukaryotic cells, are a cellular powerhouse, which generate energy for cells in the form of adenosine triphosphate (ATP) [64, 65]. Emerging evidence indicates that mitochondria play a crucial role in cellular development and function, including growth, differentiation, proliferation, and metabolism [66]. In neurodegenerative diseases, the accumulated toxic misfolded proteins and many neurotoxins damage the mitochondria in neurons and microglia [67]. There is a growing body of evidence showing that mitochondrial dysfunction is closely associated with the development of neurodegenerative diseases [68–72]. Mechanistic studies demonstrate that mitochondrial dysfunction leads to the excessive generation of free radicals, decreased ATP levels and mitochondrial membrane potential (MMP), calcium dyshomeostasis, mitochondrial permeability transition, mtDNA mutations, and perturbed mitochondrial dynamics [67] (Figure 3). In 12-month-old APPsw and APP/PS1 mouse models of AD, mitochondrial A*β* levels are closely associated with mitochondrial dysfunction and cognitive impairment [73]. In addition, mutant APP and A*β* enter mitochondria and interact with mitochondrial-related proteins, then disrupt the electron transport chain (ETC) and induce the generation of ROS, and decrease the cellular ATP levels [74, 75]. In PD, neurotoxins, such as MPTP, rotenone, and paraquat, induce dopaminergic neuronal death through the direct inhibition of the activity of mitochondrial complex I [76, 77]. In the brain of HD patients, the activity of the respiratory chain complexes is decreased, which was accompanied by the abnormal mitochondrial morphology [78]. In addition, the postmortem brain samples of HD patients exhibit impaired mitochondrial complexes II, III, and IV of the ETC [79]. Moreover, mtDNA oxidative damage-mediated impaired complex I is reported to contribute to the pathogenicity of MS [72]. The mitochondrial antioxidant defence system including SOD and catalase plays important role in clearing the endogenous free radicals effectively. In AD and familial and sporadic ALS patients, the expression level of mitochondrial SOD is decreased [80]. Therefore, maintenance of the normal function of mitochondria and the discovery of targeted drugs can effectively mitigate the progress of neurodegenerative diseases.

The article "Dietary Plant Polyphenols as the Potential Drugs in Neurodegenerative Diseases: Current Evidence, Advances, and Opportunities" was published in 2022. Journal: Oxid Med Cell Longev.

### 2.4. DNA Damage

Deoxyribonucleic acid (DNA), an important genetic material in cells, functions as the passer of genetic information with high fidelity. Otherwise, the cells undergo senescence and death when the DNA is damaged and cannot be repaired effectively. Therefore, DNA damage is implicated in various diseases, such as cancer, ageing, and neurodegenerative diseases [81–83]. There is a growing body of studies showing that DNA damage or defective DNA repair system is recognized to be a shared pathogenic mechanism, which is closely associated with the development of neurodegenerative diseases [84] (Figure 3). Oxidative DNA, DNA strand breaks, and DNA damage response (DDR) are the main lesions in neurodegenerative diseases [85, 86]. Among them, oxidative stress is especially sensitive to DNA damage and has attracted increasing attention. The high metabolic rate and high ROS levels decrease the ratio of antioxidant to prooxidant enzymes and induce oxidative stress [87]. It is reported that the base excision repair (BER) pathway consisting of DNA glycosylase changes with ageing in neurodegenerative diseases, which is primarily involved in the repair of oxidative lesions. In the brain of AD, the expressions of mitochondrial uracil DNA glycosylase and betaOGG1 glycosylase are found to be decreased [87]. At the same time, elevated DNA strand breaks, the reduced expression of DNA double-strand breaks (DSBs), repair proteins including the DNA-dependent protein kinase catalytic subunit (DNA-PKcs) and Mre11-Rad50-Nbs1 (MRN) complex proteins, and the activity of BER are identified in AD patients [88, 89]. In addition, the increased levels of oxidative lesions and single-strand breaks (SSBs) lead to serious damage of mtDNA in the neurons of ALS and PD [90, 91]. Furthermore, HD patient fibroblasts exhibit DNA oxidative lesions because the DNA repair system is impaired by mHtt [92]. Taken together, inhibition of DNA damage and the discovery of drugs that can repair DNA damage are important therapeutic strategies for neurodegenerative diseases.

### 2.5. Excitotoxicity

Excitotoxicity is a process that is triggered by the activation of the glutamate receptors owing to the pathologically high neurotransmitters such as glutamate, *α*-amino-3-hydroxy-5-methyl-4-isoxazolepropionic acid (AMPA), or N-methyl-D-aspartic acid (NMDA). Under excitotoxicity, the dendrites become degenerated and nerve cells undergo damage or even death (Figure 4). Therefore, excitotoxicity acting as a common pathogenic mechanism plays a key role in the development of various neurodegenerative diseases. Glutamate and aspartate are two major neurotransmitters that are widely distributed in neurons located in the cerebral cortex and hippocampus. They play important roles in regulating memory and learning functions. Emerging evidence indicates that the glutamate receptor is overactivated by excitatory amino acids, which damages neurons via multiple ways, including the impairment of calcium buffering, generation of free radicals, activation of the mitochondrial permeability transition (MPT), and its resultant secondary excitotoxicity [93]. The overexpression of NMDA or AMPA-type glutamate receptors is reported to induce neuronal apoptosis in vivo and in vitro [94]. In addition, the expression of NMDA receptors (NMDARs) is closely associated with mitochondrial activity, and NMDAR agonists lead to mitochondrial toxin-induced striatal damage [95]. For example, kynurenic acid (KA) and quinolinic acid (QA) induce neuronal apoptosis via activating the nuclear factor kappa B (NF-*κ*B) signaling pathway and upregulating the expressions of p53 and c-Myc [96, 97]. At present, the excitotoxicity hypothesis has been widely studied in the molecular mechanism of HD. In addition to neuronal death and neuroinflammation, mHtt is also reported to enhance the activity of NMDAR and disturb the calcium signaling pathway, ultimately leading to neuronal death [98]. Further study revealed that mHtt activates NMDAR via the postsynaptic density protein- (PSD-) 95 [99] and NR1A/NR2B known as the main NMDAR subtype in neostriatal medium-size spiny neurons [100]. In addition, the early cognitive deficit is paralleled with the activation of glutamatergic signaling in AD [101]. Emerging evidence shows that glutamate- or A*β*-induced oxidative stress and the generation of lipid peroxidation are closely associated with the activation of NMDAR in hippocampal neurons [102]. In PD, Parkin is reported to regulate the function and stability of excitatory glutamatergic synapses, while the knockdown of Parkin or overexpression of mutant Parkin results in the proliferation of glutamatergic synapses and excitotoxicity [103]. MK-801, a noncompetitive antagonist of NMDAR, is demonstrated to inhibit MPTP-induced excitotoxicity in dopaminergic neurons [104]. Therefore, neuronal excitotoxicity plays an important role in the progression of neurodegenerative diseases, while inhibitors of excitotoxicity have become promising candidates for the treatment of neurodegenerative diseases.

The article "Dietary Plant Polyphenols as the Potential Drugs in Neurodegenerative Diseases: Current Evidence, Advances, and Opportunities" was published in 2022. Journal: Oxid Med Cell Longev.

### 2.6. Biometal Dyshomeostasis

In general, metals are divided into essential and nonessential metals according to the human body needs. The essential metals include chromium, iron (Fe), copper (Cu), manganese (Mn), calcium (Ca), and zinc (Zn). They act as cofactors of enzymes to regulate cellular bioactivity. Although essential metals are important for the function of the human body, they are usually present in trace amounts. Emerging evidence indicates that essential metals exert important physiological functions in different regions of the brain, while the deficiency of essential metals in the brain commonly results in the abnormal biological process and promotes the progression of neurodegenerative diseases [105–107]. At the same time, the overaccumulation of metals in the brain also induces various detrimental events, such as oxidative damage, mitochondrial dysfunction, protein misfolding, autophagy dysfunction, neuronal death, and neuroinflammation. Therefore, intracellular metal dyshomeostasis is implicated in various neurodegenerative diseases [108, 109]. In AD, abnormal or excessive Ca released from the endoplasmic reticulum (ER) results in the disruption of intracellular Ca dyshomeostasis and ultimately leads to memory loss and cognitive dysfunction [110]. In addition, metals, including Zn, Cu, and Fe, are reported to promote A*β* aggregation and induce oxidative stress. Meanwhile, Cu accumulated in neurofibrillary tangles (NFTs) binds to Tau protein and accelerates the aggregation of Tau in vitro [111, 112]. In 6-OHDA- or MPTP-induced animal models of PD, the content of iron in the brain is found to be increased [113], and the accumulated iron leads to the degeneration and ferroptosis of nigrostriatal dopaminergic neurons [114]. In addition, Mn inhibits glycolysis and energy metabolism, which ultimately results in excitotoxicity and dysregulation of cytoskeletal integrity in YAC128Q mice, an animal model of HD [115]. Furthermore, the aberrant copper-protein interaction also promotes the progression of HD by modulating the huntingtin structure and interfering with brain lactate-energy metabolism [116]. In ALS, lead (Pb) and selenium (Se) are demonstrated to be the common risks [117, 118]. In addition, Zn and Cu acting as cofactors for SOD1 contribute to the progression of ALS [119]. Therefore, biometal homeostasis plays an important role in CNS, while the imbalance of biometals will accelerate the development of neurodegenerative diseases.

The article "Dietary Plant Polyphenols as the Potential Drugs in Neurodegenerative Diseases: Current Evidence, Advances, and Opportunities" was published in 2022. Journal: Oxid Med Cell Longev.

### 2.7. Neurotrophic Impairment

Neurotrophins are important regulators for the survival, development, function, and plasticity of neurons [120]. In general, neurotrophic factors are grouped into three major families, including neurotrophins, glia cell-line-derived neurotrophic factor (GDNF), and neurokinins. The neurotrophins are further subdivided into nerve growth factor (NGF), brain-derived neurotrophic factor (BDNF), GDNF, neurotrophin-3 (NT-3), and neurotrophin-4. There is a growing body of evidence indicating that these neurotrophic factors inhibit cell death and improve neuronal proliferation and maturation, as well as enhance the growth and function of cholinergic and dopaminergic neurons [121, 122], while neurotrophic impairment contributes to the pathogenesis of neurodegenerative diseases [123]. Among them, BDNF, a key neurotrophic factor, regulates cell death and survival of neurons via multiple signaling pathways including c-Jun N-terminal kinase (JNK), Ras homolog gene family member (RhoA), NF-*κ*B, mitogen-activated protein kinase (MAPK), phosphatidylinositol 3-kinase/protein kinase B (PI3K/Akt), and phospholipase C-*γ* (PLC-*γ*) (Figure 5). In AD, changes in the level of neurotrophic factors including BDNF, NGF, and GDNF are closely associated with the development of disease [124]. Among them, NGF is recognized as a key neurotrophic factor for the development of the cholinergic system [125]. In addition, neurotrophic factor alterations are observed in many preclinical and clinical cases of PD [126]. For example, decreased levels of BDNF in the dopaminergic area were demonstrated to be associated with the progression of PD [127]. Furthermore, GDNF, another important neurotrophic factor, is reported to play an important role in the regulation of the survival, differentiation, and maintenance of motor and dopaminergic neurons [128]. In HD, intracerebral transplantation of BDNF-overexpressing human neural stem cells promotes the migration, differentiation, and functional recovery of neurons in the unilateral QA-lesioned striatum of HD rat [129]. In addition, ciliary neurotrophic factor (CNTF) improves motor function and survival, decreases neuronal degeneration and muscle atrophy in the wobbler mouse model of ALS. In the SOD1G93A mice, tumor necrosis factor *α*- (TNF-*α*-) triggered GDNF is found to limit the degeneration of motor neurons and slow down the progression of disease [130]. Taken together, neurotrophic impairment is a key mechanism in neurodegenerative diseases, and the maintenance of normal levels of neurotrophic factors in neurons is a promising strategy for the treatment of neurodegenerative diseases.

The article "Dietary Plant Polyphenols as the Potential Drugs in Neurodegenerative Diseases: Current Evidence, Advances, and Opportunities" was published in 2022. Journal: Oxid Med Cell Longev.

### 2.8. Neuroinflammatory Responses

Microglia, the resident immune cells in the brain, play a key role in maintaining brain homeostasis and constitute the first line of defence against brain intrusion and lesions. The chronic activation of microglia under the stimulation of DAMPs/PAMPs induces the proinflammatory response and releases multiple proinflammatory mediators, including cytokines, prostaglandins, and chemokines, which are found to be elevated in the cerebrospinal fluid (CSF) and postmortem brain tissue [131] (Figure 1). Recently, inflammasome-mediated neuroinflammation has been implicated in various neurodegenerative diseases [132]. Among them, NLRP3 is the most common and well-studied inflammasome, which is implicated in the pathological development of neurodegenerative diseases [133]. In A*β*-induced BV-2 cells and APP/PS1 mice, the NLRP3 inflammasome is activated and amounts of proinflammatory cytokines including IL-1*β*, IL-6, IL-18, and TNF-*α* are subsequently secreted, which are accompanied by the cognitive decline and memory loss of APP/PS1 mice [134]. In addition, microglia are also overactivated, and the proinflammatory responses are induced in MPTP-induced PD mice [135]. Moreover, mHtt-induced abnormal activation of microglia is found to be correlated with the severity of disease in midstate HD patients [136, 137]. The mechanistic study finds that the NF-*κ*B signaling pathway is activated by mHtt, and the proinflammatory cytokines such as IL-6 and IL-8 are released [138]. In the TDP-43-overexpressed brain of LPS-treated mice, the microglia and astrocytes are overactivated. Meanwhile, the permeability of BBB is vulnerable under the stimulation of proinflammatory responses [139]. Therefore, neuroinflammation has been an important indicator of pathological development, which is implicated in various neurodegenerative diseases, and the discovery of drugs targeting the inhibition of neuroinflammation is useful for the treatment of neurodegenerative diseases.

The article "Dietary Plant Polyphenols as the Potential Drugs in Neurodegenerative Diseases: Current Evidence, Advances, and Opportunities" was published in 2022. Journal: Oxid Med Cell Longev.

## 3. The Potential Treatment of Dietary Plant Polyphenols for Neurodegenerative Diseases

Polyphenols are mainly from rich natural resources and are characterized by the presence of large multiples of phenol structural units. In general, most of the polyphenols are commonly found in dietary plants, such as the seed or skin of fruits (e.g., grape, litchi, rambutan, mangosteen, and pitahaya), vegetables (e.g., legumes, cereals, and cauliflower), various kinds of tea leaves, and also many medical herbs (e.g., *Scutellaria baicalensis*, ginkgo leaves, and *Lycium barbarum*) [140]. Emerging evidence indicates that polyphenols exhibit multiple bioactivities, including antioxidation, clearance of free radicals, anticancer, anti-inflammation, cardiovascular protection, brain protection, and prevention of obesity and diabetes. It is worth noting that most of the polyphenols manifest potential therapeutic effects in the in vitro and in vivo models of neurodegenerative diseases. However, the poor stability and low bioavailability largely limit their neuroprotective effects [141]. In this review, we summarized the neuroprotective effect and molecular mechanism of the most reported and representative polyphenols (Table 2) and the natural dietary plants enriching polyphenols in various neurodegenerative diseases (Table 3). Meanwhile, we also discussed the barricades and possibilities for polyphenols from bench to bedside.

### 3.1. Polyphenols

To date, there are thousands of polyphenols identified from natural dietary plants. In general, polyphenols are mainly classified into flavonoids and nonflavonoids. According to the hydroxylation mode and oxidation state, the flavonoids are subdivided into flavanols, flavanones, anthocyanins, flavonols, flavones, and isoflavones, while the nonflavonoids mainly include phenolic acids, phenolic alcohols, stilbenes, lignans, curcuminoids, and coumarins (Figure 6) [142].

The article "Dietary Plant Polyphenols as the Potential Drugs in Neurodegenerative Diseases: Current Evidence, Advances, and Opportunities" was published in 2022. Journal: Oxid Med Cell Longev.

#### 3.1.1. Flavonoids

Flavonoids are a large group of plant polyphenolic metabolites. They are commonly found in a variety of diets, including fruits and vegetables. Structurally, most flavonoids share a 1,2-diphenylpropane or 1,3-diphenylpropane (C6-C3-C6) skeleton [143]. In general, flavonoids are classified into 12 major types according to their chemical structures. Among them, the representative compounds of flavonols, flavanones, anthocyanins, flavonols, flavones, and isoflavones are the most common and widely reported polyphenols. The representative compounds include kaempferol, quercetin, galangin, myricetin, liquiritigenin, matteucinol, hesperidin, and naringenin; pelargonidin, rosinidin, malvidin, cyanidin, procyanidins, epicatechin, and catechin; and baicalein, apigenin, luteolin, chrysin formononetin, biochanin A, genistein, and daidzein. Several studies show that these flavonoids exert a potent neuroprotective effect in various neurodegenerative diseases via antioxidant, antiapoptosis, and anti-inflammatory responses.

*(1) Quercetin*. Quercetin, also known as 3,3′,4′,5,7-pentahydroxyflavone, belongs to flavonols. It is widely found in fruits and vegetables, such as apples, berries, onions, and capers [144]. Therefore, quercetin is recognized to be safe and displays various biological and health-promoting effects. To date, several studies indicate that quercetin protects against neurodegenerative diseases through multiple mechanisms, such as inhibition of the aggregation of misfolded proteins [145], antioxidative stress [146], and anti-inflammatory responses [147]. In APP695-transfected SH-SY5Y cells, quercetin not only exhibits antiamyloidogenic and fibril-disaggregating effects but also reduces the cytotoxicity and oxidative stress [145]. Meanwhile, quercetin decreases the levels of lactate dehydrogenase (LDH), acetylcholinesterase (AChE), and malondialdehyde (MDA), while increasing the protein levels of SOD, GSH-Px, plasma levels of catalase (CAT), and total antioxidant capacity (T-AOC) in A*β*_25-35_-induced PC-12 cells via the sirtuin1/Nrf2/HO-1 pathway [148]. It is reported that beta-secretase-1 (BACE-1) plays an important role in the generation of A*β* fragments, while quercetin can inhibit the activity of the BACE-1 enzyme through the formation of hydrogen bonds with BACE-1 [149]. In triple transgenic AD (3xTg-AD) mice, quercetin significantly decreases the protein expressions of extracellular A*β* and Tau and inhibits the proinflammatory responses in the hippocampus and amygdala, which is manifested by improvements in cognitive and behavioural function. In addition, quercetin inhibits the hyperphosphorylation of Tau, oxidative stress, and apoptosis in okadaic acid- (OA-) induced PC-12 cells via the PI3K/Akt/GSK3*β*, MAPKs, and NF-*κ*B signaling pathways [150]. In multiple PD toxin (e.g., 6-OHDA, MPTP, and rotenone)-induced nerve cells and animals, quercetin exerts potent neuroprotective effect [135]. For example, quercetin protects MN9D cells against 6-OHDA-induced neurotoxicity and reverses behavioural deficits, striatal dopamine depletion, and the loss of tyrosine hydroxylase (TH) neuronal cells in MitoPark transgenic mice. The mechanistic study found that the protein kinase D1- (PKD1-) Akt pathway is activated by quercetin [151]. In addition, quercetin attenuates rotenone-induced behavioural impairment and oxidative stress [152]. Most importantly, the combination of quercetin with piperine shows superior neuroprotective effects in antioxidative and anti-inflammatory in rotenone- and iron supplement-induced rats [153] and also in MPTP-induced rats [154]. In neuro-2a cells transiently transfected with 16Q huntingtin (Htt) and 150 Htt, quercetin increases cell viability and clears the mHtt aggregates via the upregulation of UPS activity [155]. In addition, quercetin binds to the SOD1 dimer, then blocks its fibrillization, and reduces the cytotoxicity of SOD1 fibrils in ALS [156, 157]. Emerging evidence indicates that the excessive accumulation of metal ions generates amounts of ROS levels and induces neurotoxicity, which favours the pathological process in various neurodegenerative diseases [158–160], while the treatment of quercetin improves the viability and inhibits the proinflammatory responses via inhibiting the production of ROS levels and its resultant apoptosis [161, 162]. Taken together, quercetin shows a potent neuroprotective effect in neurodegenerative diseases. However, its narrow therapeutic window, low bioavailability, and poor solubility limit its clinical application [163–165]. Thus, the structure and formulation modifications are required for quercetin to further increase its neuroprotective effect.

*(2) Hesperidin*. Hesperidin is a flavanone glycoside that exists in fruits including orange and lemon [166]. Emerging studies indicate that hesperidin possesses multiple neuroprotective activities, including the inhibition of oxidative damage [167], the suppression of neuroinflammation [168], and antiapoptosis [168]. For instance, in A*β*_1-42_-injected mice and A*β*_1-42_/LPS-induced BV-2 or HT22 cells, hesperidin exhibits potent neuroprotective effects mainly involving the inhibition of oxidative stress, antineuroinflammation, and antiapoptosis. Meanwhile, it also improves cognitive function via the Nrf2/HO-1 and TLR4/NF-*κ*B signaling pathways [167, 168]. In addition, hesperidin inhibits H_2_O_2_-induced oxidative stress via regulating the ER and TrkA signaling pathways [169] and inhibits LPS-induced apoptosis via increasing Bcl-2 protein levels and reducing the expression of phosphorylated-c-Jun N-terminal kinases (p-JNK), Bax, and caspase-3 [168]. In the 6-OHDA-induced mouse model of PD, hesperidin reduces the degeneration of DA neurons in the substantia nigra pars compacta (SNpc) via preventing mitochondrial dysfunction and inhibiting the activity of caspase-3 and caspase-9 [170]. In addition, hesperidin attenuates iron-induced mortality, oxidative stress, and mitochondrial dysfunction and restores DA levels in the Drosophila melanogaster model of PD [170]. 3-Nitropropionic acid (3-NP), an inhibitor of succinate dehydrogenase, is commonly used to induce an animal model of HD. The treatment of hesperidin can inhibit 3-NP-induced neurotoxicity and attenuate oxidative stress, dysfunction of mitochondrial complex enzymes, and locomotor activity [171]. Furthermore, hesperidin also inhibits neuroinflammation as revealed by the increased production of IL-10 and transforming growth factor- (TGF-) *β* in the mouse model of MS [172]. Regarding the permeability of hesperidin through the BBB [173], hesperidin is believed to be a promising compound for the treatment of neurodegenerative diseases.

*(3) Anthocyanins*. Anthocyanins, a type of water-soluble flavonoid, are widely found in many coloured fruits and vegetables, including blueberries, cherries, raspberries, purple grapes, and blackcurrants [174]. Thus, anthocyanins as our daily diet are safe for the human body [175]. To date, there are many bioactive anthocyanins identified, mainly including cyanidin, malvidin, delphinidin, and pelargonidin. Anthocyanins are reported to exert a neuroprotective effect in vitro and in vivo, including the inhibition of A*β* [176], the attenuation of oxidative damage [177], and the suppression of inflammatory responses [178]. In A*β*-induced HT22 cell and rat models of AD, anthocyanins restore cell viability, increasing the MMP and the level of intracellular free Ca^2+^. Meanwhile, anthocyanins decrease the protein expressions of Bax, caspase-3, caspase-9, A*β*, APP, P-Tau, and BACE-1 [179]. Anthocyanins including anthocyanoside, malvidin, and malvidin-3-O-glucoside isolated from Vaccinium myrtillus are demonstrated to inhibit the formation of A*β*_1-42_ and A*β*_1-40_ fibrils in neuro-2a cells [180, 181]. Besides, anthocyanins attenuate glutamate-induced oxidative stress via increasing the levels of GSH and GSSG and stimulating the expression of endogenous Nrf2 and HO-1 [182]. At the same time, anthocyanins inhibit glutamate-induced mitochondrial depolarization and ROS generation via reducing the intracellular Ca^2+^ levels [183]. In amyloid-beta oligomer- (A*β*O-) induced HT22 cells, anthocyanins reduce neurotoxicity via regulating PI3K/Akt/Nrf2 signaling pathways [184]. In addition, anthocyanins inhibit LPS-induced expression of NO and PGE2 and suppress the production of proinflammatory cytokines including TNF-*α* and IL-1*β* in BV-2 cells via the NF-*κ*B and Akt/MAPK signaling pathways [178]. Protocatechuic acid, a major metabolite of anthocyanin, is reported to inhibit the aggregations of A*β* and *α*-synuclein and ultimately recovers the cell viability of PC-12 cells [185]. In addition, protocatechuic acid also lessens the severity of pathological symptoms and slows down the progression of disease in the mouse model of ALS [186]. Moreover, the ability of anthocyanins to cross the BBB suggests that anthocyanins may be a promising drug for the treatment of neurodegenerative diseases [187]. Although studies indicate that anthocyanins possess potential therapeutic effects on certain neurodegenerative diseases, the effect of anthocyanins on more models of neurodegenerative diseases needs to be further confirmed and explored.

*(4) Epigallocatechin-3-Gallate*. Epigallocatechin-3-gallate (EGCG), the major component in green tea, belongs to tea polyphenols and exhibits various biological activities in the CNS [188], including antioxidative stress [189], metal-chelating ability [190], the inhibition of neuroinflammatory responses [191], and antiapoptosis [192]. In LPS-induced peripheral mononuclear blood cells (PBMCs), EGCG decreases the production of inflammatory cytokines, including TNF-*α*, IL-1*β*, and IL-6 [193]. Meanwhile, EGCG attenuates the expressions of A*β* and APP in the hippocampal neurons of D-galactose-induced AD mice [194]. Additionally, EGCG effectively remodels the structure of fibrillated amyloid proteins including *α*-synuclein and A*β* into nontoxic aggregations [195]. Through chelation with iron, EGCG reduces the expressions of iron-regulated APP and A*β* in Chinese hamster ovary cells, which are overexpressed with the APP “Swedish” mutation [196]. In A*β*-induced EOC 13.31 microglia, EGCG inhibits the neuroinflammatory responses by decreasing the expressions of TNF*α*, IL-1*β*, IL-6, and iNOS via negatively regulating the ROS-mediated NF-*κ*B pathway and activating the Nrf2/HO-1 pathway [197]. Moreover, the anti-inflammatory effect of EGCG is validated in APP/PS1 mice as evidenced by the inactivation of NLRP3 and caspase-11-dependent inflammasome via the TLR4/NF-*κ*B pathway [191]. In addition, EGCG protects PC-12 cells against H_2_O_2_- or A*β*-induced apoptosis through activating the PI3K/Akt pathway and inhibiting the GSK-3 pathway [198]. Therefore, this evidence suggests that EGCG has the potential to be developed into a new drug in the prevention and treatment of neurodegenerative diseases.

*(5) Apigenin*. Apigenin, known as 4′,5,7-trihydroxyflavone, belongs to the flavones and is widely found in common fruits and vegetables, such as parsley, celery, oranges, and grapefruit, particularly abundant in the chamomile plant [199]. Emerging evidence indicates that apigenin exerts a neuroprotective effect, including the inhibition of misfolded proteins [200], antineuroinflammation [201, 202], and antioxidant effects [203]. In the APP/PS1 mouse model of AD, apigenin reduces the A*β* plaque burden, inhibits oxidative stress, and improves memory impairment via the ERK/CREB/BDNF pathway [204]. In addition, apigenin is proven to improve learning and memory abilities in A*β*_25-35_-induced amnesic mice. Meanwhile, apigenin also reduces oxidative damage, suppresses the activity of AChE, and increases the levels of BDNF, TrkB, and phospho-CREB [205]. In chronic unpredictable mild stress- (CUMS-) induced rats, apigenin inhibits oxidative stress, upregulates PPAR*γ* expression, and suppresses the activation of NLRP3 inflammasome and the subsequent production of IL-1*β* and IL-18 [206]. In addition, apigenin inhibits the aggregation of *α*-synuclein and increases the expression of TH and dopamine D2 receptors in the rotenone-induced rat model of PD [200]. Meanwhile, apigenin protects dopaminergic neurons against oxidative injury, inhibits microglial activation, and enhances the levels of TH and BDNF in the MPTP-induced mouse model of PD [207]. Although the present studies suggest the neuroprotective effect of apigenin in AD and PD, the bioavailability, absorption, and metabolism of apigenin in vivo remain unclear [208]. Therefore, further studies associated with its pharmacokinetic parameters are still needed to be explored, which help the development of apigenin as a new drug for the treatment of neurodegenerative diseases.

*(6) Genistein*. In soybeans, isoflavones are the major component, which is reported to alleviate A*β*_1-42_-induced impairment of learning and memory ability via regulating the RAGE/LRP-1 pathway in Wistar rats [209]. Genistein, a polyphonic compound of soy isoflavones, has been reported to exert a neuroprotective effect in various neurodegenerative diseases, such as AD and PD [210, 211]. For instance, genistein improves A*β*-triggered cognitive impairment and scavenges the free radicals in vivo [210]. Meanwhile, genistein blocks the hyperphosphorylation of Tau by reducing the intracellular Ca^2+^ levels and promoting its autophagic clearance [210]. The mechanistic study indicates that genistein decreases the intracellular Ca^2+^ levels through activating the calcium/calmodulin-dependent protein kinase IV (CAMK4) [212]. In addition, genistein inhibits ischemic oxidative damage and improves behavioural deficits via the eNOS/Nrf2/HO-1 signaling pathway [213] and also protects cerebrovascular endothelial cells against A*β*_25-35_-induced oxidative damage via activating the Nrf2 and PI3K pathways [214]. In 6-OHDA-induced rat models of Parkinsonism (P) and Parkinsonism+ovariectomized (OP), genistein effectively improves spatial learning and memory impairment [211]. Furthermore, the oral genistein administration also reduces the neuronal demyelination and inhibits the secretion of IFN-*γ*, IL-12, and TNF-*α* in the splenocyte and brain of the early phase of experimental allergic encephalomyelitis (EAE) mouse, a relevant model of MS [215]. Collectively, genistein as the major component in soybeans is safe and exhibits the potential component beneficial effect in neurodegenerative diseases.

The article "Dietary Plant Polyphenols as the Potential Drugs in Neurodegenerative Diseases: Current Evidence, Advances, and Opportunities" was published in 2022. Journal: Oxid Med Cell Longev.

#### 3.1.2. Phenolic Acids

Phenolic acids usually refer to the phenolic compounds with a carboxylic acid group on the benzene ring. They are mainly divided into hydroxybenzoic acid and hydroxycinnamic acid. Phenolic acids usually exist in the binding form of amides, esters, or glycosides in a variety of dietary plants, such as plant seeds, fruit peels, and vegetable leaves. Numerous studies show that this type of polyphenols is potential therapeutic value in neurodegenerative diseases [216].

*(1) Gallic Acid*. Gallic acid, also known as 3,4,5-trihydroxy benzoic acid, belongs to hydroxybenzoic acid and is found in a variety of plants including grape seed, rose flowers, sumac, oak, and witch hazel [217]. In general, gallic acid exists in the free state of ester derivatives and polymers via the hydrolysis of terpenoids and polyphenol tannins [218]. A mounting body of researches shows that gallic acid exhibits the inhibition of misfolded proteins [219], antioxidant [219], and anti-inflammatory [220] effect in various models of neurodegenerative diseases [221]. For example, gallic acid is identified to be the most active component in grape seed extract that inhibits the formation of *κ*-CN fibrils and reduced the toxicity of *κ*-CN in PC-12 cells [222]. Meanwhile, gallic acid also inhibits the expression of A*β* protein, reduces the activity of BACE-1, inhibits neuroinflammation, and stabilizes the oxidative stress in the brain, ultimately attenuating the impaired learning and memory of APP/PS1 mice [219]. In addition, gallic acid acting as a histone acetyltransferase inhibitor decreases LPS- or A*β*-induced NF-*κ*B acetylation and cytokine production in BV-2 and primary microglia cells and Institute of Cancer Research (ICR) mice, thereby effectively inhibiting the neuroinflammation and neuronal cell death [220]. At the same time, gallic acid severing as a free radical scavenger prevents lipid peroxidation, reduces ROS levels, and increases the expression of SOD1 and GPx1 in APP/PS1 mice and AlCl_3_-induced Wistar rats [219]. In 6-OHDA-induced SH-SY5Y cells, gallic acid ameliorates the disruption of MMP, reduces the level of ROS, and inhibits apoptosis or cell death through activating the TrkB/CREB/BDNF and AKT/Keap1/Nrf2 signaling pathways [223]. In vivo, gallic acid is demonstrated to counteract oxidative stress by increasing the contents of total thiol and GPx and decreasing the levels of MDA in the hippocampus and striatum tissues of 6-OHDA-induced Wistar rats [224, 225]. In the AlCl_3_-induced Wistar rat model of ALS, gallic acid effectively improves learning ability and motor coordination via improving the antioxidant status, preventing glutamate excitotoxicity, inhibiting caspase-3 activation, and decreasing the production of proinflammatory cytokines [226]. The molecular docking analysis and in silico analysis predicted that gallic acid is a novel agonist of aryl hydrocarbon receptor (Ahr). It can inhibit the proinflammatory responses and increase the level of transforming growth factor-*β* (TGF-*β*) in EAE mice [227]. Although a large number of studies show that gallic acid has therapeutic effects on a variety of neurodegenerative diseases through multiple pathways, further researches are required to investigate its safety and effectiveness in clinical.

*(2) Chlorogenic Acid*. Chlorogenic acid (CGA), known as 3,4′,5-trihydroxy-stilbene, is the most abundant isomer of caffeoylquinic acid, which belongs to hydroxycinnamic acid and is rich in the dietary fruits and vegetable [228]. Numerous studies indicate that CGA exerts a neuroprotective effect including anti-inflammatory responses [229], antioxidative stress [230], antiapoptosis [231] and the inhibition of misfolded proteins [232, 233]. In A*β*-induced SH-SY5Y cells and APP/PS1 mice, CGA can promote the activity of lysosomes and restore the autophagic flux in the brain cells, thereby improving cognitive impairments via the mTOR/TFEB signaling pathway [232]. Besides, CGA inhibits apoptosis, improves the antioxidant capacity, and inhibits mitochondrial injury in A*β*-induced hippocampal neurons [231]. In the Tet-Off system, which controls the cytotoxicity of *α*-synuclein, CGA significantly inhibits the oxidation of dopamine and the interaction of oxidized dopamine with *α*-synuclein and degrades the oligomerization of *α*-synuclein in PC-12 cells [233]. In addition, CGA inhibits oxidative stress and ERS by reducing the expression levels of C/EBP homologous protein (CHOP) and GRP94. Meanwhile, CGA also inhibits the apoptosis in 6-OHDA-induced SH-SY5Y cells [230]. In vivo, CGA is validated to reverse motor dysfunction via enhancing the activity of antioxidant enzymes including SOD and GSH-Px in the striatum of 6-OHDA-induced Sprague-Dawley male rats [230]. Furthermore, CGA alleviates the MPTP-induced PD symptoms of mice through the anti-inflammatory and antioxidant mechanisms, which mainly involves the increased activity of SOD and CAT, decreased release of TNF-*α*, IL-1*β*, and NO, and the increased secretion of IL-10 via the NF-*κ*B signaling pathway [234]. It is reported that mitochondrial-mediated apoptotic senescence of DA neurons is implicated in MPTP-intoxicated PD mouse, while the treatment of CGA can inhibit the ratio of Bax/Bcl-2 and caspase-3 activation, which is associated with the downregulation of GSK3*β* via activating the Akt/ERK signaling pathway [235, 236]. Taken together, numerous studies are suggesting that CGA exhibits considerable protective effects in various neurodegenerative diseases. However, further efforts such as the modification of the formulation and the improvement of stability are required to push forward its clinical use.

The article "Dietary Plant Polyphenols as the Potential Drugs in Neurodegenerative Diseases: Current Evidence, Advances, and Opportunities" was published in 2022. Journal: Oxid Med Cell Longev.

#### 3.1.3. Hydroxytyrosol

At present, 30 different phenolic compounds, including oleacein, tyrosol and hydroxytyrosol, were identified from olive oil. Olive oil is the most important resource in the Mediterranean region, which has been associated with many health benefits [237–239]. The pharmacological studies show that olive oil phenols exhibit neuroprotective effects in various neurodegenerative diseases such as AD [240], PD [241], and HD [242].

Among these polyphenols, hydroxytyrosol belonging to phenolic alcohol is also found in diverse vegetable species and exerts powerful antioxidant and anti-inflammatory effect [243, 244]. Most importantly, hydroxytyrosol is able to pass through the BBB [245]. As far as we know, mitochondrial dysfunction is one of the key cellular hallmarks of neurodegenerative diseases [246]. In the 7PA2 cell cellular model simulating A*β* toxicity of AD, hydroxytyrosol can restore the energy deficiency to maintain mitochondrial function [247]. Meanwhile, hydroxytyrosol ameliorates the neuronal impairment in APP/PS1 mice via modulating mitochondrial oxidative stress, neuroinflammation, and apoptosis [248]. In addition, the treatment of hydroxytyrosol increases the cell viability in A*β*_25-35_-treated astrocytes via improving insulin sensitivity and restoring insulin signal transduction [249]. In 1-methyl-4-phenylpyridinium (MPP(+))-induced rat model of PD, hydroxytyrosol and its derivatives decrease lipid fluorescence products (LFP) and increase striatal dopamine levels and brain GSH/GSSG ratio, as well as inhibit the monoamine oxidase (MAO) isoforms and prevent neurotoxicity [250, 251]. In addition, hydroxytyrosol is demonstrated to inhibit the enzymatic and spontaneous oxidation of endogenous dopamine in PC-12 cells with MAO inhibition [252]. Moreover, it has been shown that the combination of hydroxytyrosol with donepezil which forms a novel hydroxytyrosol-donepezil hybrid has potential neuroprotective effect compared to drug alone [243]. In summary, the neuroprotective effects of olive oil phenols such as hydroxytyrosol have been determined, but the mechanisms behind these effects need to be further elucidated.

The article "Dietary Plant Polyphenols as the Potential Drugs in Neurodegenerative Diseases: Current Evidence, Advances, and Opportunities" was published in 2022. Journal: Oxid Med Cell Longev.

#### 3.1.4. Resveratrol

Stilbenes belong to natural polyphenols in which two phenyl parts are connected by the methylene of two carbon. Structurally, stilbenes are characterized by the replacement of two benzene rings with hydroxyl and methoxy groups. In general, stilbenes are not as common as other polyphenols, which exist in some plants in the form of glycosylation [142].

Resveratrol, known as 3,4,5-trihydroxystilbene, belongs to stilbenes, which is widely investigated and found to be abundant in dietary plants, including grapes, raspberries, mulberries, and peanuts [253]. Increasing studies suggest that resveratrol exerts antiageing and neuroprotective effects [254–257]. At present, the phase II clinical trials of resveratrol for AD patients are ongoing [258]. In 3xTg-AD mice, resveratrol improves memory loss and brain pathology as evidenced by the reduced protein expressions of A*β* and P-Tau in the hippocampus. The mechanism mainly involves the enhancement of proteostasis, the increased level of amyloid-degrading enzyme neprilysin, the reduced activity of BACE-1, and the increased activity of proteasome [259]. In addition to the degradation via the proteasome, the production and aggregation of A*β* are also reduced by resveratrol via direct binding to A*β* peptide [260] and autophagy induction [261]. Moreover, resveratrol promotes the insulin-degrading enzyme- (IDE-) dependent degradation of A*β*_42_ monomer and its fragments [262]. In addition, the upregulation of SIRT1 and downregulation of CD147 by resveratrol are closely associated with the abrogation of hypoxia-induced upregulation of exosomal A*β* [263, 264]. In intracerebroventricularly injected A*β* mice and A*β*-induced activation of microglia, resveratrol significantly inhibits the activation of NLRP3 inflammasome and reduces the release of proinflammatory cytokines, including IL-6, TNF-*α*, and IL-1*β*, which ultimately alleviates the learning and cognitive decline of mice [265–267]. In addition, resveratrol exerts antioxidative effects via decreasing the intracellular levels of MDA and ROS and correspondingly increasing the levels of SOD and GSH in A*β*_1-42_-induced PC-12 cells, which is correlated with the upregulation of HO-1 expression through activating the PI3K/AKT/Nrf2 signaling pathway [268]. Furthermore, the upregulation of adenosine monophosphate-activated protein kinase (AMPK) and SIRT1 is associated with the antineuroinflammation and antioxidative stress effect of resveratrol in A*β*-induced human neural stem cells [269, 270]. In MPTP-induced PD mouse and A53T *α*-synuclein transgenic mouse, resveratrol inhibits the expression of *α*-synuclein via upregulating the level of MicroRNA-214, thereby improving the motor dysfunction [271–273]. In addition, resveratrol inhibits rotenone-induced apoptosis in SH-SY5Y cells and promotes the degradation of *α*-synuclein via the AMPK/SIRT1-mediated autophagy induction in PC-12 cells overexpressing *α*-synuclein [274]. In vivo, resveratrol attenuates oxidative damage and dopamine depletion in 6-OHDA-induced PD rats [275]. Most importantly, the combinational use of resveratrol with L-Dopa alleviates the loss of dopaminergic neurons, attenuates the activation of astrocytes, and inhibits the protein levels of Bax and caspase-3 in MPTP-induced PD mice, which is more superior than resveratrol or L-Dopa alone [276]. In multiple models of HD, including the PC-12/HttQ103 cell line, Drosophila expressing mutant Httex1, and the R6/2 mice, resveratrol increases the survival of PC-12 cells and prolongs the lifespan of flies and R6/2 mice. Meanwhile, resveratrol alleviates the pathology of Drosophila and R6/2 mice via activating the ERK signaling pathway [277]. In addition, resveratrol protects the normal function of mitochondrial and improves the motor coordination and learning ability in YAC128 mice and N171-82Q transgenic mice through the AMPK, SIRT1, and peroxlsome proliferator-activated receptor-γ coactlvator-1α (PGC-1*α)* pathways [256, 278]. In thimerosal-induced SH-SY5Y and VSC4.1 cells overexpressing mutant SOD1-G93A, resveratrol increases the cell viability via the upregulation of SIRT1 [279, 280]. At the same time, resveratrol can prolong the lifespan of SOD1-G93A ALS mice [281]. In addition, resveratrol attenuates neuronal damage and promotes myelin regeneration via enhancing Olig1 and SIRT1 expression in cuprizone-intoxicated C57Bl/6 mice and EAE mice [282, 283]. However, another study reports that resveratrol significantly exacerbates demyelination and inflammation without neuroprotection in the EAE and Theiler's murine encephalomyelitis virus-induced demyelinating disease (TMEV-IDD) models of MS [284]. Therefore, resveratrol exhibits a potent neuroprotective effect in various neurodegenerative diseases. However, further studies about how to increase its safety and bioavailability are also required before it implements clinical trials.

The article "Dietary Plant Polyphenols as the Potential Drugs in Neurodegenerative Diseases: Current Evidence, Advances, and Opportunities" was published in 2022. Journal: Oxid Med Cell Longev.

#### 3.1.5. Schisandrin B

The lignans are formed by oxidative dimerization of two or more phenylpropane units [285]. Lignans are usually found in a wide variety of plant-based food, including grains, vegetables, and fruits in the form of aglycone, ester, or glycoside [286]. A large number of studies show that lignans such as Schisandrin B, justicidin A, and matairesinol have anti-inflammatory, antioxidant, and neuroprotective effects [36, 287]. Among them, Schisandrin B is one of the most abundant lignans presenting in the traditional Chinese medical herb Schisandra chinensis (SC) belonging to the medicine food homology (MFH) species. The modern pharmacological studies demonstrate that Schisandrin B exerts protective effects on neurodegenerative diseases through multiple pathways, including the inhibition of misfolded proteins [288], antioxidative stress [289], and the inhibition of inflammatory responses [287]. For instance, Schisandrin B protects SH-SY5Y cells against A*β*_1-42_-induced injury via increasing the mRNA and protein expressions of DNA methylation (DNMT), including DNMT3A and DNMT3B [290]. Besides, Schisandrin B significantly reduces the secretion of A*β* levels in N2A/SWE cells by inhibiting the transcription and translation of BACE-1 [288]. Meanwhile, Schisandrin B also antagonizes A*β*-mediated cell damage by decreasing the expression of vacuolar sorting 35 and APP in PC-12 cells [291]. GSK-3*β* is a key enzyme that is responsible for the hyperphosphorylation of Tau protein. It is reported that Schisandrin B increases the expression of p-GSK-3*β* (Ser9) but decreases the expressions of p-GSK-3*β* (Tyr216) and p-GSK-3*β* (Tyr279) and ultimately inhibits the activity of GSK-3*β* and the protein expression of Tau in APP/PS1 mice [292]. In the 6-OHDA-induced rat model of PD, Schisandrin B downregulates miR-34a expression and activates the Nrf2 pathway to reduce neuronal damage [293]. In addition, Schisandrin B protects differentiated PC-12 cells against paraquat- or tert-butylhydroperoxide- (tBHP-) induced oxidant injury via enhancing GSH redox cycling and cellular GSH levels [294, 295]. In 3-NP-induced PC-12 cells, Schisandrin B inhibits the ratio of necrotic and apoptotic cells through enhancing cellular glutathione redox status and ameliorating the cellular energy crisis, which is regulated by suppressing the JNK-mediated activation of pyruvate dehydrogenase (PDH) [296]. In addition, Schisandrin B alleviates neuroinflammatory responses as demonstrated by the decreased levels of proinflammatory cytokines, including NO, TNF-*α*, PGE2, IL-1*β*, and IL-6, in LPS-treated primary microglia and ICR mice via the TLR4-dependent MyD88/IKK/NF-*κ*B signaling pathway [287]. Taken together, Schisandrin B offers a promising therapeutic prospect in neurodegenerative diseases.

The article "Dietary Plant Polyphenols as the Potential Drugs in Neurodegenerative Diseases: Current Evidence, Advances, and Opportunities" was published in 2022. Journal: Oxid Med Cell Longev.

#### 3.1.6. Curcumin

Curcumin (1,7-bis[4-hydroxy-3-methoxyphenyl]-1,6-heptadiene-3,5-dione), also known as diferuloylmethane, is the major active ingredient of turmeric derived from the rhizome of Curcuma longa [297]. Accumulating lines of literatures show that curcumin possesses various neuroprotective effects, such as inhibiting the aggregation of misfolded proteins [298], chelating metal ions [299], antioxidation [300], and attenuating neuroinflammation [301]. In an early study, curcumin is demonstrated to effectively inhibit the formation of A*β* oligomers and fibrils. Meanwhile, curcumin binds plaques and reduces A*β* in the Tg2576 mouse model of AD [298]. In addition, curcumin inhibits the oligomerization of Tau and disintegrated preformed Tau filaments in vitro [302]. In the APP/PS1 transgenic mouse model of AD and LPS-stimulated BV-2 microglia, curcumin attenuates A*β*-induced neuroinflammation as evidenced by the inactivation of microglia and astrocytes and reduced production of proinflammatory cytokines via activating the activity of PPAR*γ* and inhibiting the NF-*κ*B signaling pathway [301, 303]. In addition, curcumin functionated as a metal chelator interacts with copper or iron to inhibit metal-induced A*β* aggregation and toxicity, as well as inhibits the inflammatory responses [299]. In PD, curcumin binds to *α*-synuclein oligomers and fibrils to decrease the cytotoxicity in SH-SY5Y cells [304]. In the MPP(+)-induced SH-SY5Y cell model of PD, curcumin increases cell viability as evidenced by the improvement of cell morphology. Meanwhile, curcumin also promotes cell proliferation and inhibits apoptosis via the upregulation of HSP90 protein [305]. In HD, curcumin prevents the formation of htt72Q-GFP (a Q-rich) and Het-s-GFP (a non Q-rich) aggregates in yeast, which is closely associated with the downregulation of Vps36, a component of the endosomal sorting complex required for transport (ESCRT-II) [306]. In addition, curcumin encapsulated solid lipid nanoparticles (C-SLNs) rescue mitochondrial swelling and reduce the levels of lipid peroxidation and ROS in 3-NP-treated rats [307]. In a clinical trial, ALS patients who were treated with curcumin showed a slight slowdown in disease progression and an improvement of aerobic metabolism and oxidative damage [308]. Furthermore, curcumin shows potent neuroprotective effects in antioxidants and inhibition of NLRP3 inflammasome activation [309, 310]. The formulation modification of curcumin using nanotechnology effectively is a promising strategy for the penetration of curcumin through BBB [311]. Taken together, the current evidence suggests that curcumin is a promising polyphenol for the treatment of neurodegenerative diseases.

The article "Dietary Plant Polyphenols as the Potential Drugs in Neurodegenerative Diseases: Current Evidence, Advances, and Opportunities" was published in 2022. Journal: Oxid Med Cell Longev.

#### 3.1.7. Imperatorin

Imperatorin, known as [9-(3-methyl but-2-acyloxy)-7H-furo[3,2-g]chromen-7-one] belongs to natural coumarins, which is widely found in the plants, including *Angelica dahurica*, *Glehnia littoralis*, and *Niphogeton* [312]. At present, only a few studies show that imperatorin and other coumarins possess neuroprotective effects, including antineuroinflammation and antioxidative damage [313]. In the scopolamine-induced mouse model of AD, imperatorin significantly reverses the memory impairment and reduces oxidative damage as evidenced by an increase in the activity of antioxidant enzymes (e.g., SOD, GPx, and glutathione reductase (GR)) and a decrease in the level of MDA [314]. In addition, imperatorin improves memory impairment via decreasing the levels of AChE, TNF-*α*, and IL-6 and upregulating the level of BDNF in the brain of LPS-induced mice [313]. Meanwhile, the imperatorin analogues show selective inhibition toward butyrylcholinesterase (BuChE) rather than AChE [315]. The in silico analysis using Autodock 4.2, Pre-ADMET, and molinspiration tools predicts that imperatorin is a potent inhibitor of COX-1, HO-1, and LOX-1. It exhibits low toxicity and a better ability to cross BBB [316]. Perfluorohexanesulfonate (PFHxS), one of the major perfluoroalkyl compounds, is widely distributed in environmental contaminants and reported to induce neuronal apoptosis, while the treatment of imperatorin effectively inhibits PFHxS-induced apoptosis of cerebellar granule cells (CGC) via the inhibition of NMDA receptor/intracellular calcium-mediated ERK pathway, suggesting that imperatorin may be a promising therapeutic candidate for the treatment of neurological disorders associated with neuroexcitotoxic damage [317]. However, the current studies on the neuroprotective effect of imperatorin are limited; thus, more in vivo and in vitro data and evidence are needed to confirm its neuroprotective effect and elucidate the molecular mechanism of imperatorin in neurodegenerative diseases.

The article "Dietary Plant Polyphenols as the Potential Drugs in Neurodegenerative Diseases: Current Evidence, Advances, and Opportunities" was published in 2022. Journal: Oxid Med Cell Longev.

### 3.2. Natural Materials Enriching Polyphenols

#### 3.2.1. Grape Seed

Grape (Putao in Chinese) is a kind of fruit that can be used for making wine, jam, grape juice, and jelly, while the grape seed is extracted and developed into various health products. Several studies suggest that the grape seed is rich in polyphenols mainly including procyanidin, catechin, epicatechin, gallic acid, and epicatechin gallate [321–323]. Therefore, the grape seed extract is widely reported to exhibit antioxidative, antiapoptosis, and anti-inflammatory effects in various neurodegenerative diseases [324–326]. For instance, grape seed-derived polyphenolics inhibit the production and accumulation of A*β* and reduce the level of A*β* in vitro and in vivo [327, 328]. In a transgenic Drosophila expressing human *α*-synuclein, grape seed extract scavenges oxygen free radicals and reduces the level of ROS and the production of toxic secondary products, ultimately slowing down the damage of mitochondria [329]. In addition, grape seed-derived polyphenols inhibit neuroinflammation via the NF-*κ*B signaling pathway in 6-OHDA-induced rats and also reduce the apoptosis of midbrain dopaminergic neurons by inhibiting the activity of caspase-3 [325]. In the Q93httexon1 Drosophila model of HD, the grape seed polyphenolic extract significantly improves the lifespan of drosophila, which is further confirmed in the R6/2 mice [326]. Therefore, the grape is not only a delicious fruit but also exhibits a potent neuroprotective effect.

#### 3.2.2. Tea Leaves

In most countries, especially in China and Japan, tea drinking is very popular and has become a local culture. In general, most of the tea is obtained from the leaves of different spices of *Camellia sinensis*. To date, the detailed ingredients in tea leaves have been well-elucidated and most of them are tea polyphenols, known as catechins, which account for almost 30-42% of dry tea leaves [330]. The pharmacological studies show that the total extract of tea leaves is reported to have a potent neuroprotective effect in various neurodegenerative diseases [331, 332]. For example, green tea catechin inhibits the activity of *β*- and *γ*-secretase to reduce the generation of A*β* [333]. In addition, thirty-three phenolic compounds are identified from the extract of fermented tea, and the anti-A*β* aggregation and antiapoptotic effects of three tea polyphenols, including (-)-catechin gallate (CG), (-)-epicatechin gallate (ECG), and EGCG, are confirmed [334]. In addition to green tea, other types of tea including white tea, oolong tea, and black tea also significantly inhibit the formation of A*β* aggregates and protect PC-12 cells against A*β*-induced neurotoxicity [335]. In addition, the oolong tea extract can reduce the intracellular ROS levels and increase the gene expressions of GPx, GSTs, SODs, and GAP-43, as well as improve the average neurite length in neuro-2a cells. Meanwhile, the oolong tea extract is validated to inhibit A*β*-induced paralysis, chemotaxis deficiency, and *α*-synuclein aggregation in *C. elegans* [336]. In MPTP-induced PD monkeys, green tea polyphenols alleviate motor impairment and dopaminergic neuronal injury [337]. Taken together, tea leaves as the raw materials of daily drinking are beneficial for our health and exhibit a potent neuroprotective effect in various neurodegenerative diseases; thus, tea drinking is recognized as a good habit for people to prevent neurodegenerative diseases.

The article "Dietary Plant Polyphenols as the Potential Drugs in Neurodegenerative Diseases: Current Evidence, Advances, and Opportunities" was published in 2022. Journal: Oxid Med Cell Longev.

#### 3.2.3. Litchi chinensis Seed

*Litchi chinensis* (Lizhi in Chinese), commonly known as lychee, belongs to a subtropical fruit. It is popular for its nutritional value and taste. In China, the seed of *Litchi chinensis* as TCMs is prescribed in many formulas for a long time owing to its great medicinal value [338]. The chemical studies show that the components in the seed of *Litchi chinensis* mainly are polyphenols, such as rutin, gallic acid, procyanidin B2, gallocatechin, epicatechin, and epicatechin-3-gallate [339]. In our research group, a purified active fraction named lychee seed fraction enriching polyphenol (LSP) is obtained from lychee seed and its neuroprotective effect is investigated in multiple models of AD [340]. For example, LSP inhibits neuronal apoptosis and improves cognitive function in PC-12 cells [341] and A*β*_25–35_-injected rats [342, 343]. In addition, LSP effectively reduces the levels of glucose, insulin, A*β*, advanced glycation end products (AGEs), and Tau in a streptozotocin- (STZ-) induced rat model of type II diabetes mellitus (T2DM) [344]. In dexamethasone- (DXM-) induced HepG2 and HT22 cells, LSP significantly improves insulin resistance (IR) and inhibits Tau proteins via the IRS-1/PI3K/Akt/GSK-3*β* pathway. Meanwhile, polyphenols including catechin, procyanidin A1, and procyanidin A2 are identified to be the bioactive components [345]. Furthermore, LSP inhibits neuroinflammation via the NF-*κ*B pathway in A*β*_1-42_-induced BV-2 cells [346], and catechin and proanthocyanidins A2 are identified to be the active components [338]. As is known to us, NLRP3 inflammasome-mediated inflammation plays an important role in neurodegenerative diseases, while autophagy negatively regulates the activation of NLRP3 inflammasome. Our recent studies demonstrate that LSP inhibits A*β*_1-42_-induced activation of NLRP3 inflammasome via autophagy induction in vitro and in vivo [340, 347]. Endoplasmic reticulum stress (ERS) is related to protein misfolding and contributes to the development of neurodegenerative diseases [348]. Oligomerized lychee fruit-derived polyphenol (OLFP) is reported to reduce the ERS in nerve cells via upregulating the mRNA expression of Wolfram syndrome-1 (Wfs1) in SAMP8 mice [349]. Although *Litchi chinensis* seed exhibits a potential therapeutic effect in AD, its effects on other neurodegenerative diseases are still unknown and need to be further investigated in the future.

The article "Dietary Plant Polyphenols as the Potential Drugs in Neurodegenerative Diseases: Current Evidence, Advances, and Opportunities" was published in 2022. Journal: Oxid Med Cell Longev.

#### 3.2.4. Scutellaria baicalensis

*Scutellaria baicalensis* (Huangqin in Chinese) belonging to the Lamiaceae is widely used in China medicine hospitals. The bioactive products of *Scutellaria baicalensis* are mainly flavonoids, including scutellarin, wogonin, baicalin, and baicalein. The pharmacological effects of *Scutellaria baicalensis* including anti-inflammation [350], antioxidation [351], and neuroprotection [352] are widely reported. Meanwhile, numerous studies show that *Scutellaria baicalensis* extract or its derived components exhibit potent neuroprotective effects in various neurodegenerative diseases [353–355]. For instance, baicalein inhibits the aggregation of A*β* and a-synuclein, as well as slows down aggregated fibre-induced neurotoxicity [356]. The thioflavin T (ThT) assay indicates that baicalein promotes the degradation of A*β*. Meanwhile, simulation and docking studies reveal that baicalein inhibits Tau aggregation through covalent modification [357]. In addition, baicalein slows down H_2_O_2_-induced apoptosis and maintains normal mitochondrial function via regulating the expression of Bcl-2 and Bax in PC-12 cells [358]. Baicalein also attenuates ERS-induced neuronal injury via reducing the expression of CHOP, glucose-regulated protein 78 (GRP78), the cleavage of X-box binding protein-1 (XBP1) and activating transcription factor 6*α* (ATF6) and phosphorylation of eukaryotic initiation factor-2*α* (eIF2) and MAPK pathways [359]. Baicalin, another flavonoid in *Scutellaria baicalensis*, reacts with copper directly and inhibits the A*β* aggregation and oxidative stress in SH-SY5Y cells [360]. In addition, baicalin inhibits neurotoxicity via HO-1-mediated autophagy induction in the rotenone-induced rat model of PD [361]. In addition to the inhibition of neuronal death, the component in *Scutellaria baicalensis* also inhibits the overactivation of microglia and the production of proinflammatory cytokines [362]. For example, baicalein inhibits neuroinflammation by negatively regulating the NLRP3/caspase-1/GSDMD pathway in MPTP-induced mice and inhibiting the NF-*κ*B and MAPK signaling pathways in rotenone-induced rats [354, 363]. Based on the above evidence, we employed UHPLC-DAD-TOF/MS analysis after a preincubation of *Scutellaria baicalensis* extract with A*β*_1-42_ to identify the potential inhibitors of A*β* fibrillization. Finally, baicalein and baicalin are found to have the highest binding affinity with A*β*, suggesting that baicalein and baicalin are the strongest inhibitors of A*β* fibrillization in *Scutellaria baicalensis* [364]. Taken together, the above evidence suggests that *Scutellaria baicalensis* and its derived flavonoids exert a potent neuroprotective effect.

The article "Dietary Plant Polyphenols as the Potential Drugs in Neurodegenerative Diseases: Current Evidence, Advances, and Opportunities" was published in 2022. Journal: Oxid Med Cell Longev.

#### 3.2.5. Ginkgo Leaves

*Ginkgo biloba*, commonly known as the maidenhair tree, is one of the oldest living tree species. The dried green leaf of *Ginkgo biloba* is a popular supplement and is commonly used in the treatment of early-stage AD [365], PD [366], and HD [367]. In the aluminum-induced rat model of AD, ginkgo leaves derived polyphenols reduce the accumulation of A*β* and improve the symptoms of AD rats via the upregulation of heat shock proteins (HSPs) [368]. In addition, ginkgo leaf extract exerts antioxidative effects via reducing the levels of ROS and RNS and increasing the contents of total superoxide dismutase (T-SOD), CAT, and GSH-Px in APPswe-expressing neuro-2a cells [369]. At the same time, the ginkgo leaf extract also inhibits H_2_O_2_-induced apoptosis via blocking the p53 pathway and reducing Bax/Bcl-2 ratio in SK-N-BE neuroblastoma cells [370]. Ginkgolic acid, a polyphenic compound, is reported to activate autophagy and clear *α*-synuclein aggregates in potassium chloride-induced SH-SY5Y cells [366]. In addition, ginkgo leaf extract can degrade poly-Q protein by increasing the activity of the proteasome via the Keap1/Nrf2 pathway [367]. Furthermore, emerging studies show that ginkgo leaf extract inhibits A*β*_1-42_-induced neuroinflammatory responses via the P38 MAPK pathway in BV-2 microglial cells [371]. Therefore, ginkgo leaf polyphenols are demonstrated to be safe and have medical value in the prevention and treatment of neurodegenerative diseases. At present, ginkgo leaf extract has been developed into a top-selling herbal supplement.

#### 3.2.6. Lycium Fruits

Lycium fruits from the plant *Lycium barbarum* (Gouqi in Chinese) are commonly been used as traditional medicine and food supplement in China for a long history. It is a traditional homology of medicine and food in Chinese medicine. The chemical studies show that Lycium fruits are rich in polysaccharides, tea polyphenols, caffeic acid, chlorogenic acid, ferulic acid, and anthocyanin [372, 373]. Although numerous studies show that polysaccharides exert potent neuroprotective effects, there are still many reports about the polyphenols and extract of Lycium fruits in various neurodegenerative diseases [374, 375]. In fibrillar A*β*_1-42_ or A*β*_25-35_ fragment induced primary rat cortical neurons, pretreatment with *Lycium barbarum* extract inhibits the release of LDH and the activity of caspase-3 via the JNK pathway [376]. In addition, the pretreatment of the alkaline extract of *Lycium barbarum* attenuates A*β*-induced apoptosis and neuronal cell death via activating the AKT pathway [377]. In vivo, *Lycium barbarum* extract significantly reduces the level of A*β*_1–42_ in hippocampal tissue and improves the learning and memory ability of APP/PS1 mice [378]. In glutamate-induced PC-12 cells, *Lycium barbarum* extract markedly increases cell viability and decreases the release of LDH, Ca^2+^ overload, ROS generation, and cell apoptosis [379]. In addition, Lycium fruit polyphenols also inhibit the level of intracellular ROS and decrease the expression of caspase-3/-8/-9 in H_2_O_2_-induced PC-12 cells [380]. Furthermore, *Lycium barbarum* extract significantly attenuates the intracellular ROS accumulation and MMP loss and increases the total levels of GSH in MPP(+)-induced PC-12 cells [381]. Therefore, both polysaccharides and polyphenols are two kinds of components in *Lycium barbarum* contributing to neuroprotection in various neurodegenerative diseases.

The article "Dietary Plant Polyphenols as the Potential Drugs in Neurodegenerative Diseases: Current Evidence, Advances, and Opportunities" was published in 2022. Journal: Oxid Med Cell Longev.

## 4. Indirect Beneficial Effect of Plant Polyphenols on Neurodegenerative Diseases

BBB is the barrier between plasma and brain cells formed by the walls of brain capillaries and glial cells and the barrier between plasma and CSF formed by the choroid plexus [382]. Extensive tight junctions are essential to maintain the integrity of the BBB, making it difficult for macromolecules and nonlipid soluble molecules to pass through [383]. Small molecules and fat-soluble substances can cross the BBB by passive diffusion and selective active transport, such as various nutrients, water, ions, organic anions, amino acids, and macromolecules (glucose) [384]. At the same time, BBB prevents the invasion of microorganisms and toxins in circulating blood to damage brain tissues. Therefore, the BBB has important biological significance for maintaining the basic stability of the internal environment of brain tissues and the normal physiological state of the CNS [385]. However, the presence of the BBB severely prevents most drugs such as many polyphenols from entering the brain to exert their effects [386].

Although a large number of studies have shown that some plant polyphenols can cross the BBB and reach the brain to exert a neuroprotective effect, there are still many polyphenols reported having indirect beneficial effects in neurodegenerative diseases [387–389]. There is growing evidence of stronger two-way communication between the gut and the brain through the neural, endocrine, and immune systems, called the brain-gut axis [390]. The gut microbiota refers to the multiple microorganisms that have coevolved in the human gut, such as symbiotic bacteria, viruses, fungi, and protozoa, which maintain homeostasis in the host by regulating digestion, immunity, metabolism, and various neurological functions. Recent studies have shown a tight association between dysbiosis of the intestinal flora and several neurodegenerative diseases, such as AD and PD [391]. Therefore, targeting regulation of the intestinal microbiota is an important strategy for the treatment of neurodegenerative diseases [389]. For example, it has been found that curcumin plays a neuroprotective role by affecting intestinal microorganisms [392]. Specifically, curcumin improves the cognition of APP/PS1 mice via altering the abundance of key bacterial species associated with AD, including *Prevotella* and *Bacteroides* [392–395]. Meanwhile, the intestinal microorganisms produce active metabolites such as demethylcurcumin and bisdemethoxycurcumin via transforming curcumin, which indirectly enhances the neuroprotective effect of curcumin [396, 397]. In addition, reduced cerebral blood flow is one of the common early features of AD, and the strict control of cardiovascular risk factors can reduce the risk of developing dementia. Therefore, the regulation of cerebral perfusion is recognized as another indirect pathway that is crucial to regulating brain function [389]. Clinical trials have shown that polyphenols are associated with enhanced cerebral blood flow and cerebral oxygenation, thus exerting neuroprotective effects [389, 398]. For example, cocoa flavonoids and curcumin are reported to increase blood flow to the cerebral cortex, thus improving cognition [399–402]. Furthermore, metabolic disorders are associated with neurodegenerative diseases, and the improvement of metabolism is also an indirect way for the treatment of neurodegenerative diseases [389]. It has been demonstrated that lychee seed polyphenols and cocoa flavonoids have therapeutic potential for AD by improving insulin resistance [345, 399]. Taken together, these indirect protective effects of plant polyphenols on neurodegenerative diseases should not be ignored.

The article "Dietary Plant Polyphenols as the Potential Drugs in Neurodegenerative Diseases: Current Evidence, Advances, and Opportunities" was published in 2022. Journal: Oxid Med Cell Longev.

## 5. Clinical Study and Application of Plant Polyphenols

To date, some clinical studies have been conducted and confirmed the neuroprotective actions of plant polyphenols, such as the ability to suppress misfolded protein accumulation and neuroinflammation, the ability to protect neurons from neurotoxin damage, and the potential to promote memory, cognition, and other brain functions. For instance, resveratrol intake (200 mg/d) for 26 weeks significantly improved memory, glucose metabolism, and functional connectivity of the hippocampus in older adults compared with the placebo treatment [403]. Turner et al. conducted a randomized, double-blind, placebo-controlled trial of resveratrol and found that resveratrol with high dose is safe and well tolerated in individuals with mild-to-moderate AD [404]. In addition, the cosupplementation of piperine with resveratrol can improve the bioavailability and efficacy of resveratrol in cognition and cerebral blood flow (CBF). Meanwhile, resveratrol also can decrease CSF MMP9, modulate neuroinflammation, and induce adaptive immunity [405]. Moreover, resveratrol attenuated the decline in minimental status examination (MMSE) scores and progressive decline in CSF A*β*_40_ levels, as well as the activity of daily living (ADL) scores, but did not alter the Tau level [406]. Curcumin, another potent neuroprotective agent, can cross the BBB due to its lipophilicity. Baum et al. imposed a double-blind, placebo-controlled clinical trial on Chinese patients (*n* = 34) who presented a decline in memory and cognitive function. After the treatment of curcumin (1 g or 4 g daily) for six months, the patients exhibited almost no significant improvement in cognitive function as compared to the placebo treatment [407]. This study suggested that the low bioavailability of curcumin is the biggest issue for its use in the treatment of neurodegenerative diseases. In addition, curcumin may be helpful for the early diagnosis of AD. Cheng et al. found that magnetic nanoparticles (MNPs) made of superparamagnetic iron oxide (SPIO) conjugated with curcumin had the potential for noninvasive diagnosis of AD using magnetic resonance imaging (MRI) [408]. Moreover, a recent study examined the effect of curcumin on cognition and mood in 60 healthy adults aged 60-85. The results showed that working memory and mood were significantly improved after 4 weeks of treatment with curcumin, confirming the potential psychological and cognitive benefits of curcumin in older populations [409]. Emerging evidence indicates that EGCG can cross the BBB to increase the memory and learning ability of the ageing brain, as well as inhibit cognitive dysfunction and reduce oxidative damage [410, 411]. De la Torre et al. demonstrated that EGCG significantly reversed the cognitive deficits of patients with Down syndrome (DS) and improved memory recognition, working memory, and quality of life [412]. A double-blind, placebo-controlled, crossover investigation demonstrated that a single dose of orally administered EGCG could modulate localized CBF parameters which are not associated with changes in cognitive performance or mood in healthy humans [413]. Similarly, another double-blind, placebo-controlled crossover study found that EGCG significantly increased the overall electroencephalography (EEG) activity in different brain regions and self-rated calmness but reduced self-rated stress compared to the placebo group, suggesting that patients who supplemented with EGCG exhibited a more relaxed and attentive state [414].

The article "Dietary Plant Polyphenols as the Potential Drugs in Neurodegenerative Diseases: Current Evidence, Advances, and Opportunities" was published in 2022. Journal: Oxid Med Cell Longev.

Researches indicate that the chronic consumption of flavonoids is associated with cognitive improvement. For instance, Kean et al. imposed a randomized, double-blind, placebo-controlled trial in healthy older adults and found that the chronic daily consumption of flavanone-rich 100% orange juice over 8 weeks is beneficial for cognitive function in healthy older adults [415]. In addition, the consumption of hesperidin-rich orange juice could enhance objective and subjective cognition throughout 6 h in healthy middle-aged adults [416]. Moreover, Lamport et al. demonstrated that consumption of flavanone-rich citrus juice in quantities enhanced CBF in 44 healthy young adults (18–30) in an acute, randomized, single-blind, placebo-controlled, clinical study [417].

To sum up, the current clinical trials confirm the efficacy of plant dietary polyphenols in neurodegenerative diseases. However, the current evidence is still very scarce. Several reasons such as low bioavailability and poor study design may be responsible for the discrepancy between the preclinical experiment and clinical trial. Therefore, increasing attention was paid to improving the bioavailability of plant polyphenols before the clinical trials.

## 6. Bioavailability of Plant Polyphenols

A large number of studies have found that the bioavailability of plant polyphenols is relatively poor, which greatly limits their efficacy [418, 419]. For example, the bioavailability of curcumin in the brain after oral administration is very low, and the systemic available dose is less than 1% of the administered dose [419]. EGCG absorption from decaffeinated green tea administered orally is only about 0.1%–0.15% in rats and about 12–26% in mice [420]. In addition, the BBB, a physical barrier that regulates the entry of substances into the brain and ensures homeostasis in the body, is the biggest barrier for drugs entering the brain [421]. Thus, plant polyphenols are administered at doses much higher than the effective circulating concentrations in the body [420, 422]. Emerging evidence indicates that polyphenols are metabolized in the body, and the metabolites take effect actually in most cases [423]. Therefore, bioavailability emerged as an unavoidable challenge for the application and development of plant polyphenols. The absorption of plant polyphenols is mainly related to the physicochemical properties of drugs, the route of administration, the absorption environment, and so on [424, 425]. For example, the insufficient water solubility of curcumin leads to low absorption and ultimately low bioavailability [426]. Thus, nanotechnology is used to improve the solubility of curcumin, and the formation of polylactic-coglycolic acid copolymer with curcumin improved the bioavailability by 40 times compared to the administration of curcumin alone in rats [427]. In addition, nanoparticulation also significantly prolonged the retention of curcumin in the cerebral cortex and hippocampus [427]. Meanwhile, other formulation modifications, including microemulsion carriers containing surfactants, oils, and cosurfactants, are also used. The optimal formulation consisting of Capryol 90 (oil), Cremophor RH40 (surfactant), and Transcutol P aqueous solution (cosurfactant) could increase the solubility of curcumin up to 32.5 mg/mL with a 22-fold increase in bioavailability [428]. In addition, curcumin formed an amorphous solid dispersion with a matrix consisting of hydroxypropyl methylcellulose, lecithin, and isomaltose, and its bioavailability increased almost 13-fold [429]. Furthermore, the formation of complexes of polyphenols with phosphatidylcholine (PC) [430], hyaluronic acid [431], polyethylene glycol [432], and dendrimer [433] can improve the solubility and bioavailability of curcumin. For example, curcumin-PC complexes reach more than triple plasma concentrations and higher area under the curve (AUC) at the same concentrations in rats as compared to curcumin alone [430]. Meanwhile, the combination of drugs also can promote the bioavailability of plant polyphenols. When EGCG was coadministered with ascorbic acid, piperine, and sucrose, respectively, the bioavailability of EGCG was significantly improved, which may be related to the inhibition of oxidative degradation of EGCG in the gastrointestinal tract, inhibition of intestinal glucuronidation, slowing down of gastrointestinal transport, and increasing retention time of EGCG [434, 435]. Distribution is the process by which drugs are absorbed and circulated in the blood to various tissues and intracellular fluids [436]. First, plant polyphenols with better fat solubility are more likely to cross the BBB and enter the brain [437]. Due to its lipophilic nature, curcumin can easily cross the BBB [438]. Metabolism refers to the chemical structural transformation of drugs [439]. After entering the body, plant polyphenols are metabolized by various enzymes, such as cytochrome P450 [440] and catechol-O-methyltransferase (COMT) [441]. After oral administration of curcumin, its glucuronide conjugates or sulfate conjugates could be detected in the blood [442]. Therefore, curcumin undergoes extensive metabolism upon arrival in the large intestine [441], which significantly affects the bioavailability and efficacy of curcumin [443].

The article "Dietary Plant Polyphenols as the Potential Drugs in Neurodegenerative Diseases: Current Evidence, Advances, and Opportunities" was published in 2022. Journal: Oxid Med Cell Longev.

Although a growing number of studies have shown that many plant polyphenols have promising effects in the treatment of neurodegenerative diseases, the low bioavailability still largely limits their neuroprotective effects. Nanoformulation is a technological system for loading and industrialization of drug molecules at the nanoscale using special carriers. Nanomodified drugs have the advantages of improving the solubility of insoluble drugs, extending the half-life of drugs, avoiding drug cytotoxicity, and increasing drug BBB permeability [444]. In this review, we made an in-depth analysis of the effect of some nanoformulations on the improvement of the bioavailability and stability of curcumin, one of the most common polyphenols, in the last decade. For instance, in curcumin-loaded lipid-PLGA nanobubbles (Cur-NBs), the solubility of curcumin was greatly increased 5-fold compared to curcumin alone [445]. In addition, curcumin-loaded PLGA nanoparticles (C-NPs) extend the half-life of curcumin and the retention time of curcumin in the cerebral cortex by 96% and in the hippocampus by 83% [427]. Curcumin delivered to nanostructured lipid carriers (NLC-Cur) has a relative lower IC_50_ of 20 *μ*g/mL and can enhance the targeting of curcumin to the brain, leading to the concentration of curcumin in vivo is 6.4-fold compared to curcumin alone [446]. In HCMEC/D3 cell monolayer permeation model, transferrin-functionalized lipid nanoparticles enhanced the BBB permeability of curcumin by 1.5-fold [447]. In addition, a lipoprotein resembling protein-free nanostructured lipid carrier (PS80-NLC) significantly enhances the affinity of curcumin with bEnd.3 cells and effectively promotes the BBB penetration and brain accumulation of curcumin [448]. Moreover, gamma scintillation studies showed that curcumin-loaded solid lipid nanoparticles (C-SLNSs) improve the brain bioavailability by 16.4 for oral administration and by 30-fold for intravenous administration compared to curcumin alone. Therefore, nanoformulations are useful tools that can improve the BBB penetration and bioavailability of plant polyphenols to exert better neuroprotective effects. However, the clinical effects of nanomodified plant polyphenols in the treatment of neurodegenerative diseases still have a long way to go.

The article "Dietary Plant Polyphenols as the Potential Drugs in Neurodegenerative Diseases: Current Evidence, Advances, and Opportunities" was published in 2022. Journal: Oxid Med Cell Longev.

## 7. Concluding Remarks and Future Perspectives

Neurodegenerative diseases are characterized by the progressive loss of the structure and function of neurons and the overactivated inflammatory responses. Emerging evidence indicates that the pathological mechanisms of neurodegenerative diseases are complicated and remain unelucidated. Commonly, the aggregation of misfolded proteins, DNA damage, mitochondrial dysfunction, oxidative stress, excitotoxicity, biometal dyshomeostasis, neurotrophic impairment, and neuroinflammatory responses are implicated in most of the neurodegenerative diseases (Figure 7). In addition, although many drugs are in clinical trials, only a small part of these drugs are successfully developed and approved for the treatment of neurodegenerative diseases. Therefore, the in-depth investigation of the mechanism and drug discovery is still essential in the future.

Polyphenols are complex plant secondary metabolites, which are mainly from dietary plants and exhibit a variety of pharmacological activities, such as antioxidant, anti-inflammatory, anticancer, liver protection, and neuroprotection [140, 449, 450]. Although most of the polyphenols are demonstrated to exhibit neuroprotective effects in various cellular and animal models, there are still very limited polyphenols or plant extracts that are developed into new drugs for the treatment of neurodegenerative diseases. In this respect, only 18 polyphenols are reported to have clinical studies by the US National Institute of Health (NIH). In addition to the poor stability, the literatures indicate that poor absorption, rapid metabolism and systemic elimination, inefficient delivery systems, and selective permeability across the BBB are also serious issues, which largely limit the bioavailability and neuroprotective effects of polyphenols in neurodegenerative diseases [451]. With the development of pharmaceutics, nanoencapsulation of polymeric nanoparticles or liposomes was employed to increase the permeability across BBB and improve the bioavailability of polyphenols. For example, an in silico validation along with the synthesis of CGA-loaded polymeric nanoparticles (CGA-NPs) by ionic gelation method is developed to overcome its pharmacological limitations and improve its stability in targeting neurodegenerative diseases [452]. In addition, liposomal resveratrol exhibits a more pronounced antioxidative effect as evidenced by the radical scavenging ability and reduction in ROS production when compared to resveratrol alone [453]. In LPS-stimulated HMC3 cells and murine acute brain slices, the liposomal curcumin shows a better effect in attenuated neuroinflammatory and reactive astrogliosis reactions than free curcumin [454]. Furthermore, the combinational use of polyphenols with other known compounds with neuroprotective effects is a promising strategy for improving their neuroprotective effects. It is reported that quercetin can function as an effective adjuvant to levodopa therapy might through its COMT/MAO inhibition property in the treatment of PD [455]. With the development of medical chemistry, increasing derivates are synthesized based on the polyphenols with the best neuroprotective effect. According to the structure of resveratrol, a series of compounds are designed and synthesized for the treatment of AD. Among them, compound 5d can be across the BBB and exhibit low toxicity in mice at doses of up to 2000 mg/kg [456]. Therefore, with the evidence suggesting the potential neuroprotective effect of polyphenols and dietary plants in various neurodegenerative diseases (Figure 7), more technologies and strategies on how to improve the absorption and stability, the modification of structure and formulation, and combination therapy are developing, which provide more opportunities from the laboratory into the clinic for polyphenols in the treatment of neurodegenerative diseases.

The article "Dietary Plant Polyphenols as the Potential Drugs in Neurodegenerative Diseases: Current Evidence, Advances, and Opportunities" was published in 2022. Journal: Oxid Med Cell Longev.

## Figures and Tables

**Figure 1:** The role of misfolded proteins in neurodegenerative diseases. The misfolded proteins, including A*β*, Tau, *α*-synuclein, and mHtt, induce the overactivation of microglia and neuronal death. The overactivated microglia release the amount of proinflammatory cytokines, including IL-6, IL-1*β*, IL-18, and TNF-*α*, and then induce neuroinflammation. Meanwhile, the overactivation of microglia aggravates the aggregation of misfolded proteins. Neuronal death was induced by misfolded proteins through multiple mechanisms, including oxidative stress, mitochondrial dysfunction, excitotoxicity, apoptosis, DNA damage, and synapse degeneration. Both neuroinflammation and neuronal death accelerate the progress of neurodegenerative diseases. However, both ALP and UPS acting as two major degradation pathways not only clear the misfolded proteins but also inhibit neuroinflammation and neuronal death in the early stage of neurodegenerative diseases. However, the overaccumulation of misfolded proteins and degenerated brain impair the normal function of ALP and UPS.

**Figure 2:** The regulation of the Keap1-Nrf2 pathway under the stimulation of ROS and electrophiles or the treatment of phenolic antioxidants in neurodegenerative diseases. Under basic conditions, Keap1, functioning as a substrate adaptor protein for Cullin3-based Cullin-RING E3 ubiquitin ligase complex around the Cullin3 (Cul3) scaffold protein, mediates the ubiquitination and proteasomal degradation of Nrf2. Under Nrf2 activation, the generated ROS or electrophiles alter the interaction between Nrf2 and its repressors under oxidative stress, resulting in the accumulation of Nrf2 in the cytoplasm and the translocation of Nrf2 into the nucleus, while the phenolic antioxidants (exogenous activator) enhance the effect of the endogenous activator on the Nrf2 pathway, thereby accelerating the dissociation of Nrf2 from Keap1 and leading to more Nrf2 translocation into the nucleus under the conditions of oxidative stress. Through the binding with Maf and ARE, Nrf2 regulates the expression of its downstream target genes, including heme oxygenase-1 (HO-1), NADPH Quinone Dehydrogenase 1 (NQO1), glutathione S-transferase (GST), glutathione peroxidase (GSH-Px), Glutamate-Cysteine Ligase Catalytic Subunit (GCLC), and superoxide dismutase (SOD). Alternatively, Nrf2 is phosphorylated by GSK-3*β*; then, *β*-transducin repeat-containing protein (*β*-TrCP) mediates its interaction with a Cul1 ubiquitin ligase complex to promote the proteasomal degradation of Nrf2, thereby inhibiting the expression of cytoprotective genes. The upregulation of cytoprotective genes prevents the generation of ROS levels, as well as oxidative damage, neuroinflammation, mitochondrial dysfunction, neuronal cell death, and protein aggregation.

The article "Dietary Plant Polyphenols as the Potential Drugs in Neurodegenerative Diseases: Current Evidence, Advances, and Opportunities" was published in 2022. Journal: Oxid Med Cell Longev.

**Figure 3:** The mitochondrial dysfunction and DNA damage in neurodegenerative diseases. The increasingly accumulated misfolded proteins (A*β*, Tau, *α*-synuclein, mHtt, *etc.*) damage the normal function of mitochondria, thus resulting in the opening of the mitochondrial permeability transition pore (MPTP). The damaged mitochondria exhibit reduced ATP levels, increased ROS generation, decreased MMP, and increased release of cytochrome c (CytoC) into the cytosol, which promotes the formation of the apoptosome and subsequent proteolytical cleavage of procaspase-3 and procaspase-7, into the activated forms. Meanwhile, the loss of MMP results in the release of apoptosis-inducing factor (AIF) that is on the cytosolic side of the outer membrane of the mitochondria into the cytosol. The activation of caspases and accumulation of AIF ultimately induce neuronal cell apoptosis. In addition, the generation of large amounts of ROS induces the production and accumulation of lipid peroxidation, which indicates that neurons undergo ferroptosis. It is worth noting that the damaged mitochondria in turn further exacerbate the aggregation of misfolded proteins. In addition, the increasingly accumulated misfolded proteins induce DNA damage in the nucleus. The damaged DNA then activates PARP-1, which catalyzes PAR formation. The free PAR translocates from the nucleus to the cytosol and mitochondria where it binds AIF, inducing AIF release from the mitochondria. Then, AIF binds the parthanatos AIF-associated nuclease (PAAN) and translocates to the nucleus and causes the generation of DNA fragmentation, which induces neuronal cell death via parthanatos.

The article "Dietary Plant Polyphenols as the Potential Drugs in Neurodegenerative Diseases: Current Evidence, Advances, and Opportunities" was published in 2022. Journal: Oxid Med Cell Longev.

**Figure 4:** The role of excitotoxicity in neurodegenerative diseases. In presynaptic neurons, glutamate (Glu) is generated through the conversion of Glutamine (Gln) with the action of glutaminase. Glu is stored in the vesicles by vesicular glutamate transporters (vGLUTs). Then, Glu is released from the vesicles and out of presynaptic neurons owing to the depolarization of the presynaptic membrane. Then, Glu binds with the ionotropic glutamate receptors (iGluRs), such as N-methyl-D-aspartate (NMDA) and *α*-amino-3-hydroxy-5-methyl-4-isoxazole propionic acid (AMPA) receptors in the postsynaptic membrane, and generates an action potential. The binding of Glu with AMPA results in Na^+^ influx and consequent membrane depolarization and opening of voltage-dependent Ca^2+^ channels (VDCC). Meanwhile, the binding of Glu with NMDA receptors (NMDARs) leads to the opening of the NMDA receptor channel under depolarizing conditions, resulting in large amounts of Ca^2+^ influx. Finally, the increased levels of cytoplasmic Ca^2+^ induce the uptake of Ca^2+^ uptake into the mitochondria, which then induces the production of reactive oxygen species (ROS) and decreases ATP levels, ultimately resulting in neuronal cell death. The excitatory amino acid transporter 3 (EAAT3) is a transporter of Glu present at the postsynaptic neuronal element. In addition, the excessively released Glu in the synaptic cleft is transported into astrocytes through the EAAT1 and EAAT2 transporters. In astrocytes, Glu is recycled and converted to Gln which is transported to neurons and converted into Glu again.

**Figure 5:** The key role of BDNF in the regulation of neuronal cell death and survival. Pre-proBDNF undergoes processing and cleavage to generate proBDNF, which is further processed to mature BDNF (mBDNF). Both proBDNF and mBDNF are stored in the proteases. ProBDNF undergoes low levels of constitutive release, while mBDNF associated with synaptic plasticity is released in an activity-dependent manner. Then, the signaling cascades are activated by the interaction of BDNF isoforms with the cell receptors located on the membrane of postsynaptic neurons, including the p75 neurotrophin receptor (p75NTR) and tropomyosin receptor kinase B (TrkB) receptor. Among them, proBDNF has a greater affinity with the p75NTR and forms the proBDNF/p75/sortilin complex, which leads to the activation of c-Jun N-terminal kinase (JNK), Ras homolog gene family member (RhoA), and nuclear factor kappa B (NF-*κ*B) signaling pathways, subsequently induces apoptosis, neuronal growth and development, and neuronal survival, respectively. In addition, mBDNF binds with TrbB and forms the mBDNF/TrkB receptor complex, which activates the following signaling pathways, including mitogen-activated protein kinase (MAPK), phosphatidylinositol 3-kinase/protein kinase B (PI3K/Akt), and phospholipase C-*γ* (PLC-*γ*). Then, the transcription factor cAMP response element-binding protein (CREB) and transcription of genes are activated. Gene modulation induces neuronal differentiation, survival, and synaptic plasticity.

The article "Dietary Plant Polyphenols as the Potential Drugs in Neurodegenerative Diseases: Current Evidence, Advances, and Opportunities" was published in 2022. Journal: Oxid Med Cell Longev.

**Figure 6:** The classification of polyphenols. Polyphenols mainly include flavonoids, phenolic acids, phenolic alcohols, stilbenes, lignans, curcuminoids, and coumarins. Flavonoids are subclassified into flavanols, flavanones, anthocyanins, flavonols, flavones, isoflavones, *etc.* Phenolic acids are divided into hydroxybenzoic acids and hydroxycinnamic acids. The representative image of plants enriching the corresponding polyphenols.

**Figure 7:** The potential treatment of natural polyphenols in neurodegenerative diseases. The natural plants especially the dietary food, such as grape, green tee, and litchi, enrich polyphenols, together with the widely reported polyphenols, such as resveratrol, curcumin, and quercetin, exhibit potent neuroprotective effects mainly involving inhibition of neuronal death and glial overactivation. The molecular mechanisms associated with the progress of neurogenerative diseases (AD, PD, HD, ALS, MS, *etc.*) include DNA damage, mitochondrial dysfunction, oxidative stress, excitotoxicity, biometal dyshomeostasis, neurotrophic impairment, neuroinflammatory responses, and the aggregation of misfolded proteins.

**Table 1:** The main current therapies and their mechanisms, effects, and limitations for neurodegenerative diseases.

Drugs	Mechanisms	Main effects	Main limitations	Diseases
Donepezil, Ralantamine, Rivastigmine	Inhibiting acetylcholinesterase	Increasing levels of synaptic acetylcholine	Increasing cognitive impairment; low CNS selectivity; gastrointestinal toxicity (nausea, vomiting, and diarrhea)	AD [18–24]
Memantine	Antagonizing N-methyl-D-aspartate-receptor (NMDAR)	Blocking glutamate from accessing NMDA receptors	Inability to slow down the progression of the disease	
Aducanumab	Human, immunoglobulin gamma 1 (IgG1) monoclonal antibody	Reducing aggregated soluble and insoluble forms of A*β*	High cost and failure to show definite effect in clinical trials	
Levodopa+Carbidopa	Inhibiting DA precursor and DOPA decarboxylase	Increasing DA levels in SNc	Wearing and movement disorders; dizziness and gastrointestinal upset	PD [25–28]
Pramipexole and Apomorphine	Agitating DA	Activating DA receptors	Less effective than levodopa; worsen dyskinesia	
Selegiline, Rasagiline, and Safinamide	Inhibiting monoamine oxidase B (MAO-B)	Preventing DA metabolism	Mild efficacy in monotherapy	
Gocovri (Amantadine)	Antivirus	Reducing levodopa-induced dyskinesia	Several side effects including psychosis, edema, constipation, and livedo reticularis	
Trihexyphenidyl	Antagonizing muscarinic acetylcholine receptor	Reducing tremor	Serious side effects including memory impairment, confusion, and hallucinations	
Levodopa+Carbidopa+Istradefylline	Inhibiting DA precursor, DOPA decarboxylase, and antagonizing A2A receptor	Reducing the “off” episodes	Higher incidence of treatment-emergent adverse events (TEAEs) and dyskinesia	
Levodopa+Carbidopa+Opicapone	Inhibiting DA precursor, DOPA decarboxylase, and catechol-o-methyl transferase (COMT)	Reducing the “off” episodes	Higher incidence of TEAEs and worsen dyskinesia than istradefylline	
Tetrabenazine (TBZ; Xenazine™) and deutetrabenazine (AUSTEDO™)	Inhibiting vesicular monoamine transporter type 2 (VMAT2)	Treating chorea associated with HD and tardive dyskinesia	Inability to slow down the progression of the disease	HD [29]
Riluzole	Blocking the presynaptic release of glutamate	Inhibiting the excitotoxicity	High cost and modest efficacy	ALS [30–33]
Edaravone (RADICAVATM)	Antioxidant	Protecting neuronal cells from oxidative stress, ameliorating motor dysfunction	Limited patient population	

The article "Dietary Plant Polyphenols as the Potential Drugs in Neurodegenerative Diseases: Current Evidence, Advances, and Opportunities" was published in 2022. Journal: Oxid Med Cell Longev.

**Table 2:** The potential effect and molecular mechanism of the representative polyphenols in various neurodegenerative diseases.

Polyphenols	Sources	Mechanisms	Models (dosage)	Diseases
Quercetin	Apples, berries, onions, and capers	Inhibition of misfolded proteins, antioxidative stress, antineuroinflammation	APP695-transfected SH-SY5Y cells (100 nM), A*β*_25-35_-induced PC-12 cells (80 *μ*M), 6-OHDA-induced MN9D cells (30 *μ*M), rotenone- and iron supplement-induced rats (50 mg/kg), MPTP-induced rats (50 mg/kg), neruo-2a cells transfected with 16Q Htt and 150 Htt (100 *μ*M), aluminum-induced rats (10 mg/kg)	AD [145, 148–150], PD [151–154, 318], HD [155], ALS [156, 157]
Hesperidin	Orange and lemon	Antineuroinflammation, antioxidative stress, antiapoptosis	A*β*_1-42_-injected mice (50 mg/kg), A*β*_1-42_/LPS-induced BV-2 or HT22 cells (50 *μ*M), H_2_O_2_-induced PC-12 cells (50 *μ*M), 3-NP-induced rats (100 mg/kg)	AD [167, 168], PD [170], HD [171], MS [172]
Anthocyanins	Blueberries, cherries, raspberries, purple grapes, and blackcurrants	Inhibition of misfolded proteins, anti-neuroinflammation, and antioxidative stress	A*β*-induced HT22 cells and rats (0.2 mg/mL and 4 mg/kg), LPS-induced BV-2 cells (100 *μ*g/mL), A*β* and *α*-synuclein-induced PC-12 cells (50 *μ*M)	AD [176, 179–181, 184, 185], PD [185], ALS [186]
Epigallocatechin-3-gallate	Green tea	Antineuroinflammation, antioxidative stress, antiapoptosis, metal-chelating ability	LPS-induced PBMCs (40 *μ*M), D-galactose-induced mice (2 mg/kg), A*β*-induced EOC 13.31 microglia (20 *μ*M), APP/PS1 mice (2 mg/kg), H_2_O_2_- or A*β*-induced PC-12 cells (200 *μ*M)	AD [191, 194, 196–198], HD [319], ALS [320]
Apigenin	Parsley, celery, oranges, and grape fruit	Inhibition of misfolded proteins, antineuroinflammation, antioxidative stress	APP/PS1 mouse (40 mg/kg), A*β*_25-35_-induced amnesic mice (20 mg/kg), rotenone-induced rats (20 mg/kg), MPTP-induced mice (20 mg/kg)	AD [204, 205], PD [200, 207]
Genistein	Soybeans	Inhibition of misfolded proteins, antineuroinflammation, antioxidative stress	EAE mice (300 mg/kg)	AD [210, 212, 214], PD [211], MS [215]
Gallic acid	Grape seed, rose flowers, sumac, oak, and witch hazel	Inhibition of misfolded proteins, antineuroinflammation, antioxidative stress	*κ*-CN fibril-induced PC-12 cells (100 *μ*M), APP/PS1 mice (20 mg/kg), LPS- and A*β*-induced BV-2 and primary microglia cells (50 *μ*M), APP/PS1 mice (20 mg/kg), 6-OHDA-induced SH-SY5Y cells (1 *μ*g/mL), 6-OHDA-induced Wistar rats (200 mg/kg), AlCl3-induced Wistar rats (200 mg/kg), EAE mice (2 mg/mouse)	AD [219, 220], PD [223–225], ALS [226], MS [227]
Chlorogenic acid	Apple, cherry, tea	Inhibition of misfolded proteins, antineuroinflammation, antioxidative stress, antiapoptosis	A*β*-induced SH-SY5Y cells (50 *μ*M), APP/PS1 mice (20 mg/kg), *α*-synuclein-induced PC-12 cells (100 *μ*M), 6-OHDA-induced SH-SY5Y cells (100 *μ*M), 6-OHDA-induced SD male rats (60 mg/kg), MPTP-induced mice (100 mg/kg)	AD [231, 232], PD [230, 233–236]
Hydroxytyrosol	Olive oil	Antineuroinflammation, antioxidative stress, antiapoptosis, and antimitochondrial dysfunction	7PA2 cells (5 *μ*M), APP/PS1 mice (5 mg/kg), A*β*_25-35_-treated astrocytes (5 *μ*M), MPP(+)-induced rat PD model (1.5 mg/kg), PC-12 cells (10 *μ*M), SHSY-5Y cells (1 *μ*M)	AD [243, 247–249], PD [250–252]
Resveratrol	Grapes, raspberries, mulberries, and peanuts	Inhibition of misfolded proteins, antineuroinflammation, antioxidative stress	3xTg-AD mice (100 mg/kg), A*β*-induced activation of microglial cells (50 nM), A*β*-induced human neural stem cells (10 *μ*M), MPTP-induced mice (50 mg/kg), A53T *α*-synuclein transgenic mouse (50 mg/kg), rotenone-induced SH-SY5Y cells (50 *μ*M), 6-OHDA-induced rats (40 mg/kg), MPTP-induced mice (10 mg/kg), YAC128 mice (1 mg/kg) and N171-82Q transgenic mice (25 mg/mouse), thimerosal-induced SH-SY5Y cells (1 *μ*M) and VSC4.1 cells (20 *μ*M), cuprizone-intoxicated C57Bl/6 mice (250 mg/kg), EAE and TMEV-IDD mice (250 mg/kg)	AD [259, 260, 263, 268–270], PD [271–276], HD [256, 277, 278], ALS [281], MS [282–284]
Schisandrin B	Schisandra chinensis	Inhibition of misfolded proteins, antineuroinflammation, antioxidative stress	A*β*_1-42_-induced SH-SY5Y cells (10 *μ*g/mL), N2A/SWE cells (10 *μ*M), A*β*-induced PC-12 cells (25 *μ*M), APP/PS1 mice (30 mg/kg), 6-OHDA-induced rats (80 mg/kg), paraquat- or tBHP-induced PC-12 cells (15 *μ*M), 3-NP-induced PC-12 cells (15 *μ*M), LPS-treated primary microglia (20 *μ*M), and ICR mice (20 mg/mL)	AD [288, 290, 292], PD [293–295], HD [296]
Curcumin	Curcuma longa	Inhibition of misfolded proteins, antineuroinflammation, antioxidative stress, chelating metal ions	Tg2576 mouse model of AD (500 mg/kg), APP/PS1 mice (150 mg/kg), LPS-stimulated BV-2 cells (20 *μ*M), MPP(+)-induced SH-SY5Y cells (40 *μ*M), ALS patients (600 mg/day)	AD [298, 299, 301, 303], PD [304, 305], HD [306, 307], ALS [308],
Imperatorin	Angelica dahurica, Glehnia littoralis, and Niphogeton	Antineuroinflammation, antioxidative stress	Scopolamine-induced mice (10 mg/kg), LPS-induced mice (10 mg/kg), PFHxS-induced cerebellar granule cells (0.5 *μ*M)	AD [314]

The article "Dietary Plant Polyphenols as the Potential Drugs in Neurodegenerative Diseases: Current Evidence, Advances, and Opportunities" was published in 2022. Journal: Oxid Med Cell Longev.

**Table 3:** The potential effect and molecular mechanism of the representative natural dietary plants in various neurodegenerative diseases.

Natural dietary plants	Components	Mechanisms	Models (dosage)	Diseases
Tea leaves	CG, ECG, and EGCG	Inhibition of misfolded proteins, antineuroinflammation, antioxidative stress, antiapoptosis	A*β*-induced PC-12 cells (150 *μ*g/mL), glutamate-induced neuro-2a and HT22 cells (25 *μ*g/mL), A*β* and *α*-synuclein aggregation in C. elegans (200 *μ*g/mL), MPTP-induced monkeys (40 mg/kg)	AD [335, 336], PD [337]
Grape seed	Procyanidin, catechin, epicatechin, gallic acid, and epicatechin gallate	Antineuroinflammation, antioxidative stress, antiapoptosis	Tg2576 mice (200 mg/kg), transgenic Drosophila expressing human *α*-synuclein (0.64 mg/100 g of culture medium), 6-OHDA-induced rats (250 mg/kg), Q93httexon1 Drosophila R6/2 mice (100 mg/kg)	AD [327, 328], PD [329, 325], HD [326]
*Litchi chinensis* seed	Rutin, gallic acid, procyanidin B2, gallocatechin, epicatechin, epicatechin-3-gallate, catechin, procyanidin A1, and procyanidin A2	Antineuroinflammation, antioxidative stress, antiapoptosis	A*β*_25–35_-induced PC-12 cells (7.60 mg/L), A*β*_25–35_-injected rats (480 mg/kg), STZ-induced rats (2.8 g/kg), DXM-induced HepG2 and HT22 cells (3.5 *μ*g/mL), A*β*_1-42_-induced BV-2 cells (10 mg/L), SAMP8 mice (100 mg/kg)	AD [341–346]
*Scutellaria baicalensis*	Scutellarin, wogonin, baicalin, baicalein	Inhibition of misfolded proteins, antineuroinflammation, antioxidative stress, antiapoptosis	H_2_O_2_-induced PC-12 cells (baicalein: 40 *μ*M), A*β*-induced SH-SY5Y cells (baicalein: 10 *μ*M), rotenone-induced rats (baicalein: 100 mg/kg), MPTP-induced mice (baicalein: 560 mg/kg)	AD [356, 357, 360, 364], PD [354, 361–363]
Ginkgo leaves	Ginkgolic acid	Inhibition of misfolded proteins, antineuroinflammation, antioxidative stress, antiapoptosis	Aluminum-induced rats (100 mg/kg), APPswe-expressing neuro-2a cells (400 *μ*g/mL), H_2_O_2_-induced SK-N-BE cells (25 *μ*g/mL), chloride-induced SH-SY5Y cells (ginkgolic acid: 80 *μ*M), A*β*_1-42_-induced BV-2 cells (90 *μ*g/mL)	AD [365, 368, 369, 371], PD [366], HD [367]
*Lycium barbarum*	Tea polyphenols, caffeic acid, chlorogenic acid, ferulic acid, and anthocyanin	Inhibition of misfolded proteins, antineuroinflammation, antioxidative stress, antiapoptosis	Fibrillar A*β*_1-42_ and A*β*_25-35_ fragments induced primary rat cortical neurons (100 *μ*g/mL), A*β*-induced neuronal cells (500 *μ*g/mL), APP/PS1 mice (10 mg/kg), glutamate-induced PC-12 cells (200 *μ*g/mL), H_2_O_2_-induced PC-12 cells (1000 *μ*g/mL)	AD [376–378]

The article "Dietary Plant Polyphenols as the Potential Drugs in Neurodegenerative Diseases: Current Evidence, Advances, and Opportunities" was published in 2022. Journal: Oxid Med Cell Longev.

## Data Availability

All data generated or analyzed in this study are available from the corresponding author on reasonable request.
